The article "Modeling the Effects of Helminth Infection on the Transmission Dynamics of Mycobacterium tuberculosis under Optimal Control Strategies" was published in 2020. Journal: Comput Math Methods Med.

# Modeling the Effects of Helminth Infection on the Transmission Dynamics of Mycobacterium tuberculosis under Optimal Control Strategies

**DOI:** 10.1155/2020/8869377

**Published:** 2020-11-17

**Authors:** Aristide G. Lambura, Gasper G. Mwanga, Livingstone Luboobi, Dmitry Kuznetsov

**Affiliations:** ^1^School of Computational and Communication Science and Engineering, The Nelson Mandela African Institution of Science and Technology, P.O. Box 447, Arusha-, Tanzania; ^2^Department of Computer Systems and Mathematics, Ardhi University, P.O. Box 35176, Dar es Salaam, Tanzania; ^3^University of Dar es Salaam, P.O. Box 2329, Dar es Salaam, Tanzania; ^4^Institute of Mathematical Sciences (IMS), Strathmore University, P.O. Box 59857-, 00200 Nairobi, Kenya

## Abstract

A deterministic mathematical model for the transmission and control of cointeraction of helminths and tuberculosis is presented, to examine the impact of helminth on tuberculosis and the effect of control strategies. The equilibrium point is established, and the effective reproduction number is computed. The disease-free equilibrium point is confirmed to be asymptotically stable whenever the effective reproduction number is less than the unit. The analysis of the effective reproduction number indicates that an increase in the helminth cases increases the tuberculosis cases, suggesting that the control of helminth infection has a positive impact on controlling the dynamics of tuberculosis. The possibility of bifurcation is investigated using the Center Manifold Theorem. Sensitivity analysis is performed to determine the effect of every parameter on the spread of the two diseases. The model is extended to incorporate control measures, and Pontryagin's Maximum Principle is applied to derive the necessary conditions for optimal control. The optimal control problem is solved numerically by the iterative scheme by considering vaccination of infants for Mtb, treatment of individuals with active tuberculosis, mass drug administration with regular antihelminthic drugs, and sanitation control strategies. The results show that a combination of educational campaign, treatment of individuals with active tuberculosis, mass drug administration, and sanitation is the most effective strategy to control helminth-Mtb coinfection. Thus, to effectively control the helminth-Mtb coinfection, we suggest to public health stakeholders to apply intervention strategies that are aimed at controlling helminth infection and the combination of vaccination of infants and treatment of individuals with active tuberculosis.

## 1. Introduction

Soil-transmitted helminth infections are common infections that affect poor communities of the world. The species that infect people are the roundworm (*Ascaris lumbricoides*), the whipworm (*Trichuris trichiura*), and the hookworm (*Necator americanus*). These parasites reside in the intestine and release eggs to contaminate the soil [1]. Approximately 1.5 billion people are infected with soil-transmitted helminths worldwide which are widely distributed in tropical and subtropical areas, with the greatest numbers occurring in sub-Saharan Africa, America, China, and East Asia [1]. On the other hand, tuberculosis (TB) is an infectious disease that is caused by the bacillus Mycobacterium tuberculosis (Mtb). Approximately 5-10% of the estimated 1.7 billion people infected with Mtb develop active TB during their lifetime [2]. The study by Watts et al. [3] suggests that infection by *trichuriasis* reduces the chance of latent tuberculosis (LTB) or blunts tuberculin skin tests (TST). Moreover, coinfection of helminth and Mtb has been a public health issue in developing countries [4]. The study by Dias et al. [5] suggests that intestinal helminth infection has a harmful effect to contain the Mtb infection and contributes to the development of active TB for coinfected individuals. Furthermore, coinfection with helminths increases the susceptibility to Mtb [6].

The article "Modeling the Effects of Helminth Infection on the Transmission Dynamics of Mycobacterium tuberculosis under Optimal Control Strategies" was published in 2020. Journal: Comput Math Methods Med.

The usefulness of mathematical modeling for understanding and assessing the dynamics of infectious diseases cannot be underrated and has been used over the years to investigate the optimal mechanisms for intervention strategies in controlling the spread of infectious diseases. The transmission and dynamics of Mtb with other diseases have been studied by many researchers [7–9]. Bhunu et al. [7] developed an HIV/AIDS and TB coinfection model that considers the treatment of exposed and active TB individuals and therapy for AIDS. They found that the treatment of exposed and active forms of TB results in stuck commencement of the AIDS stage of HIV infection. Fatmawati and Tasman [8] proposed an optimal control model for the transmission of TB-HIV coinfection. They found that the best and effective strategy to lower the TB-HIV infection is to apply a combination of anti-TB and ARV treatment. Okosun [9] discussed the synergy between malaria and schistosomiasis in the presence of treatment. Their study revealed that an effective control of malaria could be achieved if efficient treatment and prevention of schistosomiasis are implemented. There is a need for modeling coinfection of infectious diseases in areas with neglected tropical diseases (NTD) which include helminth infections, Mtb, and malaria to list a few [10], due to their geographical overlap. To the best of our understanding, no study has been carried out to consider the helminth-Mtb coinfection with the use of optimal control theory.

The article "Modeling the Effects of Helminth Infection on the Transmission Dynamics of Mycobacterium tuberculosis under Optimal Control Strategies" was published in 2020. Journal: Comput Math Methods Med.

In this paper, our emphasis is to propose a compartmental system for the codynamics of helminths and Mtb diseases and to explore the effect of helminths on Mtb and vice versa. The model is extended to incorporate four time-dependent controls, namely, educational campaign to sensitize the parents to take their babies to the Bacille Calmette-Guerin (BCG) vaccine clinic; treatment of individuals with active TB; treatment of individuals infected with helminth parasites through mass drug administration (MDA); and sanitation to lessen the ingestion rate of parasites from the polluted environment.

## 2. Materials and Methods

### 2.1. Model Formulation

The helminth-Mtb infection model is formulated under the following model assumptions:

- The susceptible individuals cannot simultaneously get infected by both diseases but rather get infected with one disease and later by the other disease
- The population is homogeneously mixed
- The incidence rate for helminth infection follows the logistic model while Mtb is assumed to be frequency-dependent
- An individual gets helminth infection after sufficient contact with the polluted environment
- Due to the fact that Mtb infection is more severe than helminth infection, we assume that coinfected individuals seek TB treatment rather than helminth infection
- The Bacille Calmette-Guerin (BCG) vaccine does not confer a total immunity

The model is formulated by considering two populations, namely, the human population and the parasite population (*M*) that are present in the contaminated environment. The human population is subdivided into nine classes, namely, susceptible (*S*), the vaccinated against Mtb (*V*_T_), those infected with Mtb but do not show clinical symptoms of TB (*E*_T_), those with active TB (*I*_T_), TB-recovered individuals (*R*_T_), those infected by helminths (*I*_H_), those who have recovered from helminths (*R*_H_), and those who are dually infected by helminths and Mtb (*I*_HT_). Thus, the total human population is given by *N* = *S* + *V*_T_ + *E*_T_ + *I*_T_ + *I*_H_ + *I*_HT_ + *R*_T_ + *R*_H_ + *R*_HT_. The susceptible population increases by recruitment through birth at the rate (1 − *η*)*bN* and by those who lose their temporary immunity against the helminths and Mtb at rates *γ*_1_ and *γ*_2_, respectively. The susceptible individuals get infected with Mtb upon sufficient contact with an infectious individual with the force of infection *λ*_T_ = (*β*_T_(*I*_T_ + *σI*_HT_))/*N*, where *β*_T_ is the transmission rate and *σ* > 1 is the modification parameter for coinfected individuals that models infectivity for susceptible individuals. The susceptible individuals also get infected by helminths after ingestion of eggs/larvae or skin penetration by infective larvae with the force of infection *λ*_H_ = *β*_H_*M*/(*K* + *M*), where *β*_H_ is the ingestion rate of parasitic worms and *K* is the density of parasites in the soil. The helminth-infected individuals increase due to susceptible individuals being infected with helminths, Mtb-vaccinated individuals infected with helminths, and coinfected individuals who recover from Mtb at the rate *τ*_2_. Furthermore, due to the fact that the BCG vaccine does not grant total protection [11], then individuals exposed to Mtb increase due to Mtb-vaccinated individuals losing their protection against Mtb and getting infected at the rate *ρλ*_T_, with *ρ* ∈ (0, 1) such that 1 − *ρ* is the efficacy of the vaccine.

The article "Modeling the Effects of Helminth Infection on the Transmission Dynamics of Mycobacterium tuberculosis under Optimal Control Strategies" was published in 2020. Journal: Comput Math Methods Med.

The chronic infection by helminths alters the chance of getting infected and the progression of coinfecting parasites (virus or bacteria) [12]; as a result, individuals infested with helminths are at higher risk of developing tuberculosis [13]. Therefore, individuals coinfected with helminth and Mtb are increased by helminth-infected individuals being infected with Mtb at the force of infection *gλ*_T_, where *g* > 1 is the modification parameter that models increased susceptibility to Mtb, and Mtb-exposed individuals getting infected by helminths at a force of infection *λ*_H_. In addition, the number of individuals with active TB increases as individuals progressed from the exposed class at the rate*k*and coinfected individuals recovered from helminth infection at the rate*τ*_1_and decreases due to natural recovery at the rate*τ*_2_. The parasite populations in the environment increase as they are released by the helminth-infected individuals at the rate *ε*_1_ and coinfected individuals at the rate *ε*_2_ and are cleared from the environment at a rate *μ*_*M*_.The description above is illustrated in Figure 1, and the governing system of nonlinear differential equations is shown in model (1). The model parameters are described in Table 1.

(1) $$\begin{array}{c} \left(\begin{array}{c} \frac{dS}{dt}=\left(1-\eta \right)bN+\gamma_{1}R_{\text{H}}+\gamma_{2}R_{\text{T}}-\left(\mu +\lambda_{\text{T}}+\lambda_{\text{H}}\right)S,\\ \frac{dV_{\text{T}}}{dt}=\eta bN-\left(\mu +\rho \lambda_{\text{T}}+\lambda_{\text{H}}\right)V_{\text{T}},\\ \frac{dE_{\text{T}}}{dt}=\lambda_{\text{T}}S+\rho \lambda_{\text{T}}V_{\text{T}}+\lambda_{\text{T}}R_{\text{H}}-\left(\mu +k+\lambda_{\text{H}}\right)E_{\text{T}},\\ \frac{dI_{\text{T}}}{dt}=kE_{\text{T}}+\tau_{1}I_{\text{HT}}-\left(\mu +d_{\text{T}}+\tau_{2}+\lambda_{\text{H}}\right)I_{\text{T}},\\ \frac{dI_{\text{H}}}{dt}=\lambda_{\text{H}}S+\lambda_{\text{H}}V_{\text{T}}+\lambda_{\text{H}}R_{\text{T}}+\tau_{2}I_{\text{HT}}-\left(g\lambda_{\text{T}}+\mu +d_{\text{H}}+\tau_{1}+\varepsilon_{1}\right)I_{\text{H}},\\ \frac{dI_{\text{HT}}}{dt}=g\lambda_{\text{T}}I_{\text{H}}+\lambda_{\text{H}}\left(E_{\text{T}}+I_{\text{T}}\right)-\left(\mu +d_{\text{HT}}+\tau_{1}+\tau_{2}+\varepsilon_{2}\right)I_{\text{HT}},\\ \frac{dR_{\text{T}}}{dt}=\tau_{2}I_{\text{T}}-\left(\lambda_{\text{H}}+\mu +\gamma_{2}\right)R_{\text{T}},\\ \frac{R_{\text{H}}}{dt}=\tau_{1}I_{\text{H}}-\left(\lambda_{\text{T}}+\mu +\gamma_{1}\right)R_{\text{H}},\\ \frac{dM}{dt}=\varepsilon_{1}I_{\text{H}}+\varepsilon_{2}I_{\text{HT}}-\mu_{M}M, \end{array}\right. \end{array}$$

where

(2) $$\begin{array}{c} \lambda_{\text{T}}=\frac{\beta_{\text{T}}\left(I_{\text{T}}+\sigma I_{\text{HT}}\right)}{N},\\ \lambda_{\text{H}}=\frac{\beta_{\text{H}}M}{M+K}. \end{array}$$

We perform a qualitative analysis of model (1) using a dimensionless version such that dimensionless variables obtained by setting *s* = *S*/*N*, *v*_T_ = *V*_T_/*N*, *e*_T_ = *E*_T_/*N*, *i*_T_ = *I*_T_/*N*, *i*_H_ = *I*_H_/*N*, *i*_HT_ = *I*_HT_/*N*, *r*_T_ = *R*_T_/*N*, *r*_H_ = *R*_H_/*N*, *r*_HT_ = *R*_HT_/*N*, and *m* = *M*/*K* replace the original variables *S*, *V*_T_, *E*_T_, *I*_T_, *I*_T_, *I*_HT_, *R*_T_, *R*_H_, *R*_HT_, and *M*, respectively, in which the rate of change of the population at time *t* is given by

(3) $$\begin{array}{c} \frac{dN}{dt}=\left(b-\mu \right)N+d_{\text{T}}I_{\text{T}}-\left(d_{\text{H}}+\varepsilon_{1}\right)I_{\text{H}}-\left(d_{\text{HT}}+\varepsilon_{2}\right)I_{\text{HT}}. \end{array}$$

Upon differentiating dimensionless variables with respect to time and using equation (3), system (1) becomes

(4) $$\begin{array}{c} \frac{ds}{dt}=\left(1-\eta \right)b+\gamma_{1}r_{\text{H}}+\gamma_{2}r_{\text{T}}-\left(b+\lambda_{\text{T}}^{*}+\lambda_{\text{H}}^{*}-d_{\text{T}}i_{\text{T}}-\left(d_{\text{H}}+\varepsilon_{1}\right)i_{\text{H}}-\left(d_{\text{HT}}+\varepsilon_{2}\right)i_{\text{HT}}\right)s,\\ \frac{dv_{\text{T}}}{dt}=\eta b-\left(b+\rho \lambda_{\text{T}}^{*}+\lambda_{\text{H}}^{*}-d_{\text{T}}i_{\text{T}}-\left(d_{\text{H}}+\varepsilon_{1}\right)i_{\text{H}}-\left(d_{\text{HT}}+\varepsilon_{2}\right)i_{\text{HT}}\right)v_{\text{T}},\\ \frac{de_{\text{T}}}{dt}=\lambda_{\text{T}}^{*}\left(s+\rho v_{\text{T}}+r_{\text{H}}\right)-\left(b+k+\lambda_{\text{H}}^{*}-d_{\text{T}}i_{\text{T}}-\left(d_{\text{H}}+\varepsilon_{1}\right)i_{\text{H}}-\left(d_{\text{HT}}+\varepsilon_{2}\right)i_{\text{HT}}\right)e_{\text{T}},\\ \frac{di_{\text{T}}}{dt}=ke_{\text{T}}+\tau_{1}i_{\text{HT}}-\left(b+d_{\text{T}}+\lambda_{\text{H}}^{*}+\tau_{2}-d_{\text{T}}i_{\text{T}}-\left(d_{\text{H}}+\varepsilon_{1}\right)i_{\text{H}}-\left(d_{\text{HT}}+\varepsilon_{2}\right)i_{\text{HT}}\right)i_{\text{T}},\\ \frac{di_{\text{H}}}{dt}=\lambda_{\text{H}}^{*}\left(s+v_{T}+r_{T}\right)+\tau_{2}i_{\text{HT}}-\left(b+d_{\text{H}}+\tau_{1}+\varepsilon_{1}+g\lambda_{\text{T}}^{*}-d_{\text{T}}i_{\text{T}}-\left(d_{\text{H}}+\varepsilon_{1}\right)i_{\text{H}}-\left(d_{\text{HT}}+\varepsilon_{2}\right)i_{\text{HT}}\right)i_{\text{H}},\\ \frac{di_{\text{HT}}}{dt}=g\lambda_{\text{T}}^{*}i_{\text{H}}+\lambda_{\text{H}}^{*}\left(e_{\text{T}}+i_{\text{T}}\right)-\left(b+\tau_{1}+\tau_{2}+\varepsilon_{2}+d_{\text{HT}}-d_{\text{T}}i_{\text{T}}-\left(d_{\text{H}}+\varepsilon_{1}\right)i_{\text{H}}-\left(d_{\text{HT}}+\varepsilon_{2}\right)i_{\text{HT}}\right)i_{\text{HT}},\\ \frac{dr_{\text{T}}}{dt}=\tau_{2}i_{\text{T}}-\left(b+\gamma_{2}+\lambda_{\text{H}}^{*}-d_{\text{T}}i_{\text{T}}-\left(d_{\text{H}}+\varepsilon_{1}\right)i_{\text{H}}-\left(d_{\text{HT}}+\varepsilon_{2}\right)i_{\text{HT}}\right)r_{\text{T}},\\ \frac{dr_{\text{H}}}{dt}=\tau_{1}i_{\text{H}}-\left(b+\gamma_{1}+\lambda_{\text{T}}^{*}-d_{\text{T}}i_{\text{T}}-\left(d_{\text{H}}+\varepsilon_{1}\right)i_{\text{H}}-\left(d_{\text{HT}}+\varepsilon_{2}\right)i_{\text{HT}}\right)r_{\text{H}},\\ \frac{dm}{dt}=\varepsilon_{1}i_{\text{H}}+\varepsilon_{2}i_{\text{HT}}-\mu_{M}m, \end{array}$$

subject to condition *s* + *v*_T_ + *e*_T_ + *i*_T_ + *i*_H_ + *i*_HT_ + *r*_T_ + *r*_H_ = 1.

The article "Modeling the Effects of Helminth Infection on the Transmission Dynamics of Mycobacterium tuberculosis under Optimal Control Strategies" was published in 2020. Journal: Comput Math Methods Med.

### 2.2. Disease-Free Equilibrium (DFE)

The DFE point of system (4) is obtained by setting the right-hand sides of the equations to zero with *e*_T_ = 0, *i*_T_ = 0, *i*_H_ = 0, *i*_HT_ = 0, *r*_T_ = 0, *r*_H_ = 0, *r*_HT_ = 0, and *m* = 0 to obtain the DFE *ℰ*_0_ = (1 − *η*, *η*, 0, 0, 0, 0, 0, 0, 0, 0).

### 2.3. Effective Reproduction Number

The principles of the next-generation matrix [22] are used to obtain the effective reproduction number.

(5) $$\begin{array}{c} R_{\text{T}}=\frac{\beta_{\text{T}}k\left(1+\eta \left(\rho -1\right)\right)}{\left(b+k\right)\left(b+d_{\text{T}}+\tau_{2}\right)}, \end{array}$$

(6) $$\begin{array}{c} R_{\text{H}}=\frac{\beta_{\text{H}}\varepsilon_{1}}{\mu_{M}\left(b+d_{\text{H}}+\varepsilon_{1}+\tau_{1}\right)}, \end{array}$$

corresponding to the reproduction numbers for the Mtb and helminth infection transmission models obtained from the positive eigenvalues of the next-generation matrix, respectively.

### 2.4. Local Stability of the Disease-Free Equilibrium

**Theorem 1 .**

The disease-free equilibrium point is locally asymptotically stable if *ℛ*_HT_ < 1 and unstable if either *ℛ*_T_ > 1 or *ℛ*_H_ > 1.

The article "Modeling the Effects of Helminth Infection on the Transmission Dynamics of Mycobacterium tuberculosis under Optimal Control Strategies" was published in 2020. Journal: Comput Math Methods Med.

**Proof**

We first obtain the Jacobian matrix at the disease-free equilibrium *ℰ*_0_ in order to prove this theorem. The Jacobian matrix is given by

(7) $$\begin{array}{c} J_{E_{0}}=\left(\begin{array}{ccccccccc} -b & 0 & 0 & l_{0} & -l_{1} & -l_{2} & \gamma_{2} & \gamma_{1} & -\beta_{\text{H}}s_{0}\\ 0 & -b & 0 & \left(\rho \beta_{\text{T}}-d_{\text{T}}\right)v_{\text{T}0} & -l_{3} & -l_{4} & 0 & 0 & -\beta_{\text{H}}v_{\text{T}0}\\ 0 & 0 & -\left(b+k\right) & \beta_{\text{T}}\left(s_{0}+\rho v_{\text{T}0}\right) & 0 & \beta_{\text{T}}\sigma \left(s_{0}+\rho v_{\text{T}0}\right) & 0 & 0 & 0\\ 0 & 0 & k & -l_{5} & 0 & \tau_{1} & 0 & 0 & 0\\ 0 & 0 & 0 & 0 & -l_{6} & \tau_{2} & 0 & 0 & \beta_{\text{H}}\\ 0 & 0 & 0 & 0 & 0 & -l_{7} & 0 & 0 & 0\\ 0 & 0 & 0 & \tau_{2} & 0 & 0 & -l_{8} & 0 & 0\\ 0 & 0 & 0 & 0 & \tau_{1} & 0 & 0 & -l_{9} & 0\\ 0 & 0 & 0 & 0 & \varepsilon_{1} & \varepsilon_{2} & 0 & 0 & -\mu_{M} \end{array}\right), \end{array}$$

where

(8) $$\begin{array}{c} l_{0}=\left(d_{\text{T}}-\beta_{\text{T}}\right)s_{0},\\ l_{1}=\left(d_{\text{H}}+\varepsilon_{1}\right)s_{0},\\ l_{2}=\left(\sigma \beta_{\text{T}}-\left(d_{\text{HT}}+\varepsilon_{2}\right)\right)s_{0},\\ l_{3}=\left(d_{\text{H}}+\varepsilon_{1}\right)v_{\text{T}0},\\ l_{4}=\left(\rho \sigma \beta_{\text{T}}-\left(d_{\text{HT}}+\varepsilon_{2}\right)\right)v_{\text{T}0},\\ l_{5}=\left(b+d_{\text{T}}+\tau_{2}\right),\\ l_{6}=\left(b+d_{\text{H}}+\tau_{1}\right),\\ l_{7}=\left(b+\tau_{1}+\tau_{2}+\varepsilon_{2}+d_{\text{HT}}\right),\\ l_{8}=\left(b+\gamma_{2}\right),\\ l_{9}=\left(b+\gamma_{1}\right). \end{array}$$

Now, the characteristic polynomial of the Jacobian matrix *J*_*ℰ*_0__ is given by

(9) $$\begin{array}{c} p\left(\lambda \right)={\left(b+\lambda \right)}^{2}\left(b+\gamma_{1}+\lambda \right)\left(b+\gamma_{2}+\lambda \right)\left(b+d_{\text{HT}}+\tau_{1}+\tau_{2}+\lambda +\varepsilon_{2}\right)\left(\lambda^{2}+\left(2b+k+d_{\text{T}}+\tau_{2}\right)\lambda +\left(b+k\right)\left(b+d_{\text{T}}+\tau_{2}\right)\left[1-R_{\text{T}}\right]\right)\left(\lambda^{2}+\left(b+d_{\text{H}}+\varepsilon_{1}+\mu_{M}+\tau_{1}\right)\lambda +\mu_{M}\left(b+d_{\text{H}}+\varepsilon_{1}+\tau_{1}\right)\left[1-R_{\text{H}}\right]\right). \end{array}$$

Clearly, from equation (9), the eigenvalues of *J*_*ℰ*_0__ are as follows: *λ*_1,2_ = −*b* < 0, *λ*_2_ = −(*b* + *γ*_1_) < 0, *λ*_3_ = −(*b* + *γ*_2_) < 0, *λ*_4_ = −(*b* + *d*_HT_ + *τ*_1_ + *τ*_2_ + *ε*_2_) < 0, and

(10) $$\begin{array}{c} \left(\lambda^{2}+\left(2b+k+d_{\text{T}}+\tau_{2}\right)\lambda +\left(b+k\right)\left(b+d_{\text{T}}+\tau_{2}\right)\left[1-R_{\text{T}}\right]\right)\left(\lambda^{2}+\left(b+d_{\text{H}}+\varepsilon_{1}+\mu_{M}+\tau_{1}\right)\lambda +\mu_{M}\left(b+d_{\text{H}}+\varepsilon_{1}+\tau_{1}\right)\left[1-R_{\text{H}}\right]\right)=0. \end{array}$$

Applying Routh-Hurwitz conditions [23] on equation (10), it has strictly negative real roots if *ℛ*_T_ < 1 and *ℛ*_H_ < 1. Thus, the DFE point *ℰ*_0_ is locally asymptotically stable whenever *ℛ*_HT_ < 1 and unstable if either *ℛ*_T_ > 1 or *ℛ*_H_ > 1.

The article "Modeling the Effects of Helminth Infection on the Transmission Dynamics of Mycobacterium tuberculosis under Optimal Control Strategies" was published in 2020. Journal: Comput Math Methods Med.

### 2.5. Global Stability of the Disease-Free Equilibrium

We investigate the global asymptotic stability of the disease-free equilibrium of model (9) by using the theory applied by Chavez et al. [24]. System (9) is written as

(11) $$\begin{array}{c} \frac{dX}{dt}=F\left(X,Y\right),\\ \frac{dY}{dt}=G\left(X,Y\right),G\left(X,0\right)=0, \end{array}$$

where *X* = (*s*, *v*_T_, *r*_T_, *r*_H_) ∈ *ℝ*_+_^4^ represents the number of uninfected individuals and *Y* = (*e*_T_, *i*_T_, *i*_H_, *i*_HT_, *m*) ∈ *ℝ*_+_^5^ represents the number of infected individuals including the latent and infectious individuals.

The DFE is given by *ℰ*_0_ = (*X*_0_^∗^, 0), where *X*_0_^∗^ = (1 − *η*, *η*). The conditions in equation (12) must be satisfied to guarantee local asymptotic stability:

(12) $$\begin{array}{c} \frac{dX}{dt}=F\left(X^{*},0\right),X^{*}\text{is}\text{globally}\text{asmptotically}\text{stable}\left(\text{g}.\text{a}.\text{s}\right),\\ G\left(X,Y\right)=BY-\hat{G}\left(X,Y\right),\text{where}\hat{G}\left(X,Y\right)\geq 0\text{for}\left(X,Y\right)\in \Sigma , \end{array}$$

and $B=D_{Y}\hat{G}\left(X^{*},0\right)$ is *M*-matrix (that is, the off-diagonal elements of matrix *B* are nonnegative); and Σ is the region where the model makes biological sense. If the equations in (4) satisfy the conditions in (12), then the following theorem holds.

**Theorem 2 .**

The fixed point *ℰ*_0_ is a globally asymptotically stable equilibrium of system (4) given that *ℛ*_HT_ < 1 and that the conditions in (12) are fulfilled.

**Proof**

System (4) as written in equation (12) can be rewritten in a reduced form:

(13) $$\begin{array}{c} {\left.\frac{dX}{dt}\right|}_{Y=0}=\left(\begin{array}{c} \left(1-\eta \right)b-bs\\ \eta b-bv_{\text{T}}\\ 0 \end{array}\right). \end{array}$$

Solving equation one in (13) gives *s*(*t*) = (1 − *η*) + (*s*_0_ − (1 − *η*))*e*^−*bt*^ implying that *s*(*t*)⟶1 − *η* as *t*⟶∞. Similarly, solving equation two in (13) gives *v*_T_(*t*) = *η* + (*v*_T0_ − *η*)*e*^−*bt*^ implying that *v*_T_(*t*)⟶*η* as *t*⟶0. Therefore, the first condition in (12) is satisfied.

Let

(14) $$\begin{array}{c} \begin{array}{c} \left(\begin{array}{c} {\hat{G}}_{1}\left(X,Y\right)\\ {\hat{G}}_{2}\left(X,Y\right)\\ {\hat{G}}_{3}\left(X,Y\right)\\ {\hat{G}}_{4}\left(X,Y\right)\\ {\hat{G}}_{5}\left(X,Y\right) \end{array}\right)=\left(\begin{array}{c} \chi_{1}\lambda_{\text{T}}^{*}\left(1-\frac{s+\rho v_{\text{T}}}{\chi_{1}}\right)-\lambda_{\text{T}}^{*}r_{\text{H}}+\lambda_{\text{H}}^{*}e_{\text{T}}-d_{\text{T}}i_{\text{T}}e_{\text{T}}-\chi_{2}i_{\text{H}}e_{\text{T}}-\chi_{3}i_{\text{HT}}e_{\text{T}}\\ \lambda_{\text{H}}^{*}i_{\text{T}}-d_{\text{T}}i_{\text{T}}^{2}-\chi_{2}i_{\text{H}}i_{\text{T}}-\chi_{3}i_{\text{HT}}i_{\text{T}}\\ \beta_{\text{H}}m\left(1-\frac{s+v_{\text{T}}+r_{\text{T}}}{1+m}\right)+g\lambda_{\text{T}}^{*}i_{\text{H}}-d_{\text{T}}i_{\text{T}}i_{\text{H}}-\chi_{2}i_{\text{H}}^{2}-\chi_{3}i_{\text{HT}}i_{\text{H}}\\ -g\lambda_{\text{T}}^{*}i_{\text{H}}-\lambda_{\text{H}}^{*}\left(e_{\text{T}}+i_{\text{T}}\right)-d_{\text{T}}i_{\text{T}}i_{\text{HT}}-\chi_{2}i_{\text{H}}i_{\text{HT}}-\chi_{3}i_{\text{HT}}^{2}\\ 0 \end{array}\right) \end{array},\\ \begin{array}{c} B=\left(\begin{array}{ccccc} -\left(b+k\right) & \beta_{\text{T}}\left(s_{0}+\rho v_{\text{T}0}\right) & 0 & \beta_{\text{T}}\sigma \left(s_{0}+\rho v_{\text{T}0}\right) & 0\\ k & -\left(b+d_{\text{T}}+\tau_{2}\right) & 0 & \tau_{1} & 0\\ 0 & 0 & -\left(b+d_{\text{H}}+\tau_{1}+\varepsilon_{1}\right) & \tau_{2} & \beta_{\text{H}}\\ 0 & 0 & 0 & -\Gamma & 0\\ 0 & 0 & \varepsilon_{1} & \varepsilon_{2} & -\mu_{M} \end{array}\right), \end{array} \end{array}$$

where *χ*_1_ = (1 + *η*(*ρ* − 1)), *χ*_2_ = *d*_H_ + *ε*_1_, *χ*_3_ = *d*_HT_+*ε*_3_, and Γ = *b* + *τ*_1_ + *τ*_2_ + *ε*_2_ + *d*_HT_. From equation (14), we observe that ${\hat{G}}_{4}\left(X,Y\right)<0$ implying that the second condition in (12) is not fulfilled, so *ℰ*_0_ may not be globally asymptotically stable. This suggests the existence of multiple equilibria.

The article "Modeling the Effects of Helminth Infection on the Transmission Dynamics of Mycobacterium tuberculosis under Optimal Control Strategies" was published in 2020. Journal: Comput Math Methods Med.

### 2.6. The Effect of Helminth Infection on Mtb and Vice Versa

We analyze the effect of helminth infection on Mtb infection and vice versa, by first expressing *ℛ*_H_ in terms of *ℛ*_T_. We solve for *b* from the expression of *ℛ*_T_ in equation (5) to get

(15) $$\begin{array}{c} b=\frac{-\theta_{1}R_{\text{T}}+\sqrt{\theta_{2}R_{\text{T}}^{2}+\theta_{3}R_{\text{T}}}}{2R_{\text{T}}}, \end{array}$$

where *θ*_1_ = *k* + *d*_T_ + *τ*_2_, *θ*_2_ = (*k* + *d*_T_ + *τ*_2_)^2^ − 4*k*(*d*_T_ + *τ*_2_), *θ*_3_ = 4*β*_T_*k*(1 + *η*(*ρ* − 1)).

Then, substituting *b* into the expression for *ℛ*_H_, we get

(16) $$\begin{array}{c} R_{\text{H}}=\frac{\beta_{\text{H}}\varepsilon_{1}}{\mu_{M}\left(\left(\left(-\theta_{1}R_{\text{T}}+\sqrt{\theta_{2}R_{\text{T}}^{2}+\theta_{3}R_{\text{T}}}\right)/2R_{\text{T}}\right)+d_{\text{H}}+\varepsilon_{1}+\tau_{1}\right)}. \end{array}$$

Differentiating equation (16) partially with respect to *ℛ*_T_ gives

(17) $$\begin{array}{c} \frac{\partial R_{\text{H}}}{\partial R_{\text{T}}}=\frac{\theta_{3}\beta_{\text{H}}\varepsilon_{1}R_{\text{T}}}{\mu_{M}\sqrt{R_{\text{T}}\left(\theta_{2}R_{\text{T}}+\theta_{3}\right)}{\left(2R_{\text{T}}\left(d_{\text{H}}+\varepsilon_{1}+\tau_{1}\right)-\theta_{1}R_{\text{T}}+\sqrt{R_{\text{T}}\left(\theta_{2}R_{\text{T}}+\theta_{3}\right)}\right)}^{2}}. \end{array}$$

Now, whenever the right-hand side of equation (17) is strictly positive, an increase in the Mtb incidence in the society results in an increase in the incidence of helminth infection in the society.

If RHS of equation (17) is equal to zero, it means that Mtb incidences have no influence on the spread of helminth infection.

Also, expressing *b* in terms of *ℛ*_H_ from the expression of *ℛ*_H_ in equation (6), we get

(18) $$\begin{array}{c} b=\frac{\beta_{\text{H}}\varepsilon_{1}-\theta_{6}R_{\text{H}}}{\mu_{M}R_{\text{H}}}, \end{array}$$

where *θ*_6_ = *μ*_*M*_(*d*_H_ + *τ*_1_). Then, expressing *ℛ*_T_ in terms of *ℛ*_H_, we have

(19) $$\begin{array}{c} R_{\text{T}}=\frac{\beta_{\text{T}}k\left(1+\eta \left(\rho -1\right)\right)\mu_{M}^{2}R_{\text{H}}^{2}}{\left(\beta_{\text{H}}\varepsilon_{1}+\left(\mu_{M}k-\theta_{6}\right)R_{\text{H}}\right)\left(\beta_{\text{H}}\varepsilon_{1}+\left(\mu_{M}\left(d_{\text{T}}+\tau_{2}\right)-\theta_{6}\right)R_{\text{H}}\right)}, \end{array}$$

Differentiating *ℛ*_T_ with respect to *ℛ*_H_, we get

(20) $$\begin{array}{c} \frac{\partial R_{\text{T}}}{\partial R_{\text{H}}}=\frac{k\varepsilon_{1}R_{\text{H}}\mu_{M}^{2}\beta_{\text{H}}\beta_{\text{T}}\left(1+\eta \left(\rho -1\right)\right)\left[R_{\text{H}}\left(\mu_{M}\left(d_{\text{T}}+k+\tau_{2}\right)-2\theta_{6}\right)+2\beta_{\text{H}}\varepsilon_{1}\right]}{{\left(R_{\text{H}}\left(k\mu_{M}-\theta_{6}\right)+\beta_{\text{H}}\varepsilon_{1}\right)}^{2}{\left(R_{\text{H}}\left(\mu_{M}\left(d_{\text{T}}+\tau_{2}\right)-\theta_{6}\right)+\beta_{\text{H}}\varepsilon_{1}\right)}^{2}}. \end{array}$$

Whenever *μ*_*M*_(*d*_T_ + *k* + *τ*_2_) ≥ 2*θ*_6_, then *∂ℛ*_T_/*∂ℛ*_H_ is strictly positive. This indicates that helminth infection incidence results in an increase in Mtb infection incidence in the society. Thus, helminth infection enhances Mtb infection in the society.

### 2.7. Existence of Backward Bifurcation

To determine the local asymptotic stability of the endemic equilibrium, we apply the Center Manifold Theorem developed by [25]. To use the theory, we make the subsequent change of variables: let *x*_1_ = *s*, *x*_2_ = *v*_T_, *x*_3_ = *e*_T_, *x*_4_ = *i*_T_, *x*_5_ = *i*_H_, *x*_6_ = *i*_HT_, *x*_7_ = *r*_T_, *x*_8_ = *r*_H_, and *x*_9_ = *m*. Then, model system (4) is often written within the following form:

(21) $$\begin{array}{c} \frac{dX}{dt}=F\left(x\right)=\left(f_{1}\left(x\right),f_{2}\left(x\right),f_{3}\left(x\right),f_{4}\left(x\right),f_{5}\left(x\right),f_{6}\left(x\right),f_{7}\left(x\right),f_{8}\left(x\right),f_{9}\left(x\right)\right) \end{array}$$

where

(22) $$\begin{array}{c} \frac{dx_{1}}{dt}=f_{1}\left(x\right)=\left(1-\eta \right)b+\gamma_{1}x_{8}+\gamma_{2}x_{7}-\left(b+\beta_{\text{T}}\left(x_{4}+\sigma x_{6}\right)-d_{\text{T}}x_{4}-\left(d_{\text{H}}+\varepsilon_{1}\right)x_{5}-\left(d_{\text{HT}}+\varepsilon_{2}\right)x_{6}\right)x_{1},\\ \frac{dx_{2}}{dt}=f_{2}\left(x\right)=\eta b-\left(b+\rho \beta_{\text{T}}\left(x_{4}+\sigma x_{6}\right)+\frac{\beta_{\text{H}}x_{9}}{1+x_{9}}-d_{\text{T}}x_{4}-\left(d_{\text{H}}+\varepsilon_{1}\right)x_{5}-\left(d_{\text{HT}}+\varepsilon_{2}\right)x_{6}\right)x_{2},\\ \frac{dx_{3}}{dt}=f_{3}\left(x\right)=\beta_{\text{T}}\left(x_{4}+\sigma x_{6}\right)\left(x_{1}+\rho x_{2}+x_{8}\right)-\left(b+k+\frac{\beta_{\text{H}}x_{9}}{1+x_{9}}-d_{\text{T}}x_{4}-\left(d_{\text{H}}+\varepsilon_{1}\right)x_{5}-\left(d_{\text{HT}}+\varepsilon_{2}\right)x_{6}\right)x_{3},\\ \frac{dx_{4}}{dt}=f_{4}\left(x\right)=kx_{3}+\tau_{1}x_{6}-\left(b+d_{\text{T}}+\tau_{2}+\frac{\beta_{\text{H}}x_{9}}{1+x_{9}}-d_{\text{T}}x_{4}-\left(d_{\text{H}}+\varepsilon_{1}\right)x_{5}-\left(d_{\text{HT}}+\varepsilon_{2}\right)x_{6}\right)x_{4},\\ \frac{dx_{5}}{dt}=f_{5}\left(x\right)=\frac{\beta_{\text{H}}x_{9}}{1+x_{9}}\left(x_{1}+x_{2}+x_{7}\right)+\tau_{2}x_{6}-\left(b+d_{\text{H}}+\tau_{1}+\varepsilon_{1}+g\beta_{\text{T}}\left(x_{4}+\sigma x_{6}\right)-d_{\text{T}}x_{4}-\left(d_{\text{H}}+\varepsilon_{1}\right)x_{5}-\left(d_{\text{HT}}+\varepsilon_{2}\right)x_{6}\right)x_{5},\\ \frac{dx_{6}}{dt}=f_{6}\left(x\right)=g\beta_{\text{T}}\left(x_{4}+\sigma x_{6}\right)x_{5}+\frac{\beta_{\text{H}}x_{9}}{1+x_{9}}\left(x_{3}+x_{4}\right)-\left(b+\tau_{1}+\tau_{2}+\varepsilon_{2}+d_{\text{HT}}-d_{\text{T}}x_{4}-\left(d_{\text{H}}+\varepsilon_{1}\right)x_{5}-\left(d_{\text{HT}}+\varepsilon_{2}\right)x_{6}\right)x_{6},\\ \frac{dx_{7}}{dt}=f_{7}\left(x\right)=\tau_{2}x_{4}-\left(b+\gamma_{2}+\frac{\beta_{\text{H}}x_{9}}{1+x_{9}}-d_{\text{T}}x_{4}-\left(d_{\text{H}}+\varepsilon_{1}\right)x_{5}-\left(d_{\text{HT}}+\varepsilon_{2}\right)x_{6}\right)x_{7},\\ \frac{dx_{8}}{dt}=f_{8}\left(x\right)=\tau_{1}x_{5}-\left(b+\gamma_{1}+\beta_{\text{T}}\left(x_{4}+\sigma x_{6}\right)-d_{\text{T}}x_{4}-\left(d_{\text{H}}+\varepsilon_{1}\right)x_{5}-\left(d_{\text{HT}}+\varepsilon_{2}\right)x_{6}\right)x_{8},\\ \frac{dx_{10}}{dt}=f_{9}\left(x\right)=\varepsilon_{1}x_{5}+\varepsilon_{2}x_{6}-\mu_{M}x_{10}. \end{array}$$

So the Jacobian matrix of system (22) at the disease-free equilibrium (*ℰ*_0_) is given by

(23) $$\begin{array}{c} \begin{array}{c} J_{E_{0}}=\left(\begin{array}{ccccccccc} -b & 0 & 0 & J_{0} & -J_{1} & -J_{2} & \gamma_{2} & \gamma_{1} & -\beta_{\text{H}}s_{0}\\ 0 & -b & 0 & \left(\rho \beta_{\text{T}}-d_{\text{T}}\right)v_{\text{T}0} & -J_{3} & -J_{4} & 0 & 0 & -\beta_{\text{H}}v_{\text{T}0}\\ 0 & 0 & -\left(b+k\right) & \beta_{\text{T}}^{*}\left(s_{0}+\rho v_{\text{T}0}\right) & 0 & \beta_{\text{T}}^{*}\sigma \left(s_{0}+\rho v_{\text{T}0}\right) & 0 & 0 & 0\\ 0 & 0 & k & -J_{5} & 0 & \tau_{1} & 0 & 0 & 0\\ 0 & 0 & 0 & 0 & -J_{6} & \tau_{2} & 0 & 0 & \beta_{\text{H}}\\ 0 & 0 & 0 & 0 & 0 & -J_{7} & 0 & 0 & 0\\ 0 & 0 & 0 & \tau_{2} & 0 & 0 & -J_{8} & 0 & 0\\ 0 & 0 & 0 & 0 & \tau_{1} & 0 & 0 & -J_{9} & 0\\ 0 & 0 & 0 & 0 & \varepsilon_{1} & \varepsilon_{2} & 0 & 0 & -\mu_{M} \end{array}\right) \end{array}, \end{array}$$

where *J*_0_ = (*d*_T_ − *β*_T_)*s*_0_, *J*_1_ = (*d*_H_ + *ε*_1_)*s*_0_, *J*_2_ = (*σβ*_T_ − (*d*_HT_ + *ε*_2_))*s*_0_, *J*_3_ = (*d*_H_ + *ε*_1_)*v*_T0_, *J*_4_ = (*ρσβ*_T_^∗^ − (*d*_HT_ + *ε*_2_))*v*_T0_, *J*_5_ = (*b* + *d*_T_ + *τ*_2_), *J*_6_ = (*b* + *d*_H_ + *τ*_1_), *J*_7_ = (*b* + *τ*_1_ + *τ*_2_ + *ε*_2_ + *d*_HT_), *J*_8_ = (*b* + *γ*_2_), and *J*_9_ = (*b* + *γ*_1_).

The article "Modeling the Effects of Helminth Infection on the Transmission Dynamics of Mycobacterium tuberculosis under Optimal Control Strategies" was published in 2020. Journal: Comput Math Methods Med.

Recall that *ℛ*_HT_ = max{*ℛ*_H_, *ℛ*_T_}. If we consider *ℛ*_HT_ = 1 (that is, *ℛ*_H_ < *ℛ*_T_ = 1), let *β*_T_ = *β*_T_^∗^ be a bifurcation parameter. Then, *ℛ*_T_ = 1 gives

(24) $$\begin{array}{c} \beta_{\text{T}}=\beta_{\text{T}}^{*}=\frac{\left(b+k\right)\left(b+d_{\text{T}}+\tau_{2}\right)}{k\left(1+\eta \left(\rho -1\right)\right)}. \end{array}$$

The Jacobian *J*_*ℰ*_0__ has a simple zero eigenvalue whose related right eigenvectors are denoted by *w* = [*w*_1_, *w*_2_, *w*_3_, *w*_4_, *w*_5_, *w*_6_, *w*_7_, *w*_8_, *w*_9_]^*T*^.where *w*_1_ = ((*J*_8_(*d*_T_ − *β*_T_^∗^)*s*_0_ + *γ*_2_*τ*_2_)/*bJ*_8_)*w*_4_ + ((*μ*_*M*_*γ*_1_*τ*_1_ − *J*_1_*J*_9_ − *β*_T_^∗^*ε*_1_*s*_0_*J*_9_)/*bμ*_*M*_*J*_9_)*w*_5_, *w*_2_ = (((*ρβ*_T_^∗^ − *d*_T_)*v*_T0_)/*b*)*w*_4_ − ((*μ*_*M*_(*d*_H_ + *ε*_1_) + *β*_H_*ε*_1_)/*bμ*_*M*_)*w*_5_, *w*_3_ = *β*_T_^∗^(*s*_0_ + *ρv*_T0_)*w*_4_/(*b* + *k*), *w*_4_ = *w*_4_ > 0, *w*_5_ = *w*_5_ > 0, *w*_6_ = 0, *w*_7_ = (*τ*_2_*w*_4_)/*J*_8_, *w*_8_ = (*τ*_1_*w*_5_)/*J*_9_, and *w*_9_ = (*ε*_1_*w*_5_)/*μ*_*M*_.

The left eigenvectors of *J*_*ℰ*_0__ associated with the simple eigenvalues are denoted by *v* = [*v*_1_, *v*_2_, *v*_3_, *v*_4_, *v*_5_, *v*_6_, *v*_7_, *v*_8_, *v*_9_]^*T*^, where *v*_1_ = *v*_2_ = *v*_7_ = *v*_8_ = 0, *v*_3_ = *kv*_4_/(*b* + *k*), *v*_4_ = *v*_4_ > 0, *v*_5_ = *v*_5_ > 0, *v*_6_ = ((*kβ*_T_^∗^*σ*(*s*_0_ + *ρv*_T0_) + *τ*_1_(*b* + *k*))/*J*_7_(*b* + *k*))*v*_4_ + ((*τ*_2_*μ*_*M*_ + *ε*_2_*β*_H_)/*J*_7_*μ*_*M*_)*v*_5_, and *v*_9_ = (*β*_H_*v*_5_)/*μ*_*M*_.

The article "Modeling the Effects of Helminth Infection on the Transmission Dynamics of Mycobacterium tuberculosis under Optimal Control Strategies" was published in 2020. Journal: Comput Math Methods Med.

The coefficients *a* and *b* that decide the local dynamics of the endemic equilibrium point are defined in equations (25) and (26):

(25) $$\begin{array}{c} a=\overset{n}{\underset{k,j,i=1}{\sum }}v_{k}w_{i}w_{j}\frac{\partial^{2}f_{k}}{\partial x_{i}\partial x_{j}}\left(E_{0},\beta_{T}^{*}\right), \end{array}$$

(26) $$\begin{array}{c} b=\overset{n}{\underset{k,i=1}{\sum }}v_{k}w_{i}\frac{\partial^{2}f_{k}}{\partial x_{i}\partial \beta_{T}^{*}}\left(E_{0},\beta_{T}^{*}\right). \end{array}$$

From system (22), the nonzero partial derivatives of *F* related to *a* at DFE are given by

(27) $$\begin{array}{c} \frac{\partial^{2}f_{1}}{\partial x_{4}\partial x_{1}}=d_{\text{T}}-\beta_{\text{T}}^{*},\\ \frac{\partial^{2}f_{1}}{\partial x_{5}\partial x_{1}}=d_{\text{H}}+\varepsilon_{1},\\ \frac{\partial^{2}f_{1}}{\partial x_{6}\partial x_{1}}=d_{\text{H}}+\varepsilon_{2}-\sigma \beta_{\text{T}}^{*},\\ \frac{\partial^{2}f_{2}}{\partial x_{4}\partial x_{2}}=d_{\text{T}}-\rho \beta_{\text{T}}^{*},\\ \frac{\partial^{2}f_{2}}{\partial x_{5}\partial x_{2}}=d_{\text{H}}+\varepsilon_{1},\\ \frac{\partial^{2}f_{2}}{\partial x_{6}\partial x_{2}}=d_{\text{HT}}+\varepsilon_{2}-\sigma \rho \beta_{\text{T}}^{*},\\ \frac{\partial^{2}f_{2}}{\partial x_{9}\partial x_{2}}=-\beta_{\text{H}},\\ \frac{\partial^{2}f_{3}}{\partial x_{4}\partial x_{3}}=d_{\text{T}},\\ \frac{\partial^{2}f_{3}}{\partial x_{5}\partial x_{3}}=d_{\text{H}}+\varepsilon_{1},\\ \frac{\partial^{2}f_{3}}{\partial x_{6}\partial x_{3}}=d_{\text{HT}}+\varepsilon_{2},\\ \frac{\partial^{2}f_{3}}{\partial x_{9}\partial x_{3}}=-\beta_{\text{H}},\\ \frac{\partial^{2}f_{3}}{\partial x_{4}\partial x_{1}}=\beta_{\text{T}},\\ \frac{\partial^{2}f_{3}}{\partial x_{6}\partial x_{1}}=\sigma \beta_{\text{T}},\\ \frac{\partial^{2}f_{3}}{\partial x_{4}\partial x_{2}}=\rho \beta_{\text{T}},\\ \frac{\partial^{2}f_{3}}{\partial x_{6}\partial x_{2}}=\rho \sigma \beta_{\text{T}},\\ \frac{\partial^{2}f_{3}}{\partial x_{4}\partial x_{8}}=\beta_{\text{T}},\\ \frac{\partial^{2}f_{3}}{\partial x_{6}\partial x_{8}}=\sigma \beta_{\text{T}},\\ \frac{\partial^{2}f_{4}}{\partial x_{4}^{2}}=d_{\text{T}},\\ \frac{\partial^{2}f_{4}}{\partial x_{5}\partial x_{4}}=d_{\text{H}}+\varepsilon_{1},\\ \frac{\partial^{2}f_{4}}{\partial x_{6}\partial x_{4}}=d_{\text{HT}}+\varepsilon_{2},\\ \frac{\partial^{2}f_{4}}{\partial x_{9}\partial x_{4}}=-\beta_{\text{H}},\\ \frac{\partial^{2}f_{5}}{\partial x_{4}\partial x_{5}}=d_{\text{T}}-g\beta_{\text{T}}^{*},\\ \frac{\partial^{2}f_{5}}{\partial x_{5}^{2}}=d_{\text{H}}+\varepsilon_{1},\\ \frac{\partial^{2}f_{5}}{\partial x_{6}\partial x_{5}}=d_{\text{HT}}+\varepsilon_{2}-g\sigma \beta_{\text{T}}^{*},\\ \frac{\partial^{2}f_{5}}{\partial x_{9}\partial x_{1}}=\beta_{\text{H}},\\ \frac{\partial^{2}f_{5}}{\partial x_{9}\partial x_{2}}=\beta_{\text{H}},\\ \frac{\partial^{2}f_{5}}{\partial x_{9}\partial x_{7}}=\beta_{\text{H}},\\ \frac{\partial^{2}f_{6}}{\partial x_{4}\partial x_{6}}=d_{\text{T}},\\ \frac{\partial^{2}f_{6}}{\partial x_{5}\partial x_{6}}=d_{\text{H}}+\varepsilon_{1}+g\sigma \beta_{\text{T}}^{*},\\ \frac{\partial^{2}f_{6}}{\partial x_{6}^{2}}=d_{\text{HT}}+\varepsilon_{2},\\ \frac{\partial^{2}f_{6}}{\partial x_{4}\partial x_{5}}=g\beta_{\text{T}}^{*},\\ \frac{\partial^{2}f_{6}}{\partial x_{9}\partial x_{3}}=\beta_{\text{H}},\\ \frac{\partial^{2}f_{6}}{\partial x_{9}\partial x_{4}}=\beta_{\text{H}},\\ \frac{\partial^{2}f_{7}}{\partial x_{9}\partial x_{7}}=-\beta_{\text{H}},\\ \frac{\partial^{2}f_{7}}{\partial x_{4}\partial x_{7}}=d_{\text{T}},\\ \frac{\partial^{2}f_{7}}{\partial x_{5}\partial x_{7}}=d_{\text{H}}+\varepsilon_{1},\\ \frac{\partial^{2}f_{7}}{\partial x_{6}\partial x_{7}}=d_{\text{HT}}+\varepsilon_{2},\\ \frac{\partial^{2}f_{8}}{\partial x_{4}\partial x_{8}}=d_{\text{T}}-\beta_{\text{T}}^{*},\\ \frac{\partial^{2}f_{8}}{\partial x_{5}\partial x_{8}}=d_{\text{H}}+\varepsilon_{1},\\ \frac{\partial^{2}f_{8}}{\partial x_{6}\partial x_{8}}=d_{\text{HT}}+\varepsilon_{2}-\sigma \beta_{\text{T}}^{*}. \end{array}$$

Therefore, equation (25) becomes

(28) $$\begin{array}{c} a=\left(\frac{a_{0}w_{4}^{2}}{b\left(b+k\right)J_{8}}+\frac{a_{1}w_{4}w_{5}}{bJ\mu_{M}J_{8}J_{9}\left(b+k\right)}\right)v_{3}+\left(d_{\text{T}}w_{4}^{2}+\frac{\left(\mu_{M}\left(d_{\text{H}}+\varepsilon_{1}\right)-\beta_{\text{H}}\varepsilon_{1}\right)}{\mu_{M}}w_{4}w_{5}\right)v_{4}+\left(\frac{a_{2}w_{4}w_{5}}{bJ_{8}\mu_{M}^{2}}+\frac{a_{3}w_{5}^{2}}{bJ_{9}\mu_{M}^{2}}\right)v_{5}+\frac{a_{4}w_{4}w_{5}}{\mu_{M}\left(b+k\right)}v_{6}, \end{array}$$

where

(29) $$\begin{array}{c} a_{0}=bd_{\text{T}}\beta_{\text{T}}^{*}J_{8}\left(s_{0}+\rho v_{\text{T}0}\right)+J_{8}\rho \beta_{\text{T}}^{*}v_{\text{T}0}\left(b+k\right)\left(\rho \beta_{\text{T}}^{*}-d_{\text{T}}\right)+\left(J_{8}\left(d_{\text{T}}-\beta_{\text{T}}^{*}\right)s_{0}+\gamma_{2}\tau_{2}\right)\sigma \beta_{\text{T}}^{*},\\ a_{1}=\beta_{\text{T}}^{*}\left(s_{0}+\rho v_{\text{T}0}\right)bJ_{8}J_{9}\left(\mu_{M}\left(d_{\text{H}}+\varepsilon_{1}\right)-\beta_{\text{H}}\varepsilon_{1}\right)+\beta_{\text{T}}^{*}\mu_{M}\left(b+k\right)\left(\sigma J_{9}\left(\mu_{M}\gamma_{1}\tau_{1}-J_{1}J_{8}-\beta_{\text{T}}^{*}\varepsilon_{1}s_{0}J_{9}\right)-b\tau_{1}J_{8}\right)-\rho \beta_{\text{T}}^{*}J_{8}J_{9}b\left(b+k\right)\left(\mu_{M}\left(d_{\text{H}}+\varepsilon_{1}\right)+\beta_{\text{H}}\varepsilon_{1}\right),\\ a_{2}=\left(d_{\text{T}}-g\beta_{\text{T}}^{*}\right)bJ_{8}\mu_{M}^{2}+\left(J_{8}\left(d_{\text{T}}-\beta_{\text{T}}^{*}\right)s_{0}+\gamma_{2}\tau_{2}\right)\varepsilon_{1}\beta_{\text{H}}\mu_{M}+b\mu_{M}\varepsilon_{1}\beta_{\text{H}}\tau_{2},\\ a_{3}=bJ_{9}\mu_{M}^{2}\left(d_{\text{H}}+\varepsilon_{1}\right)+\beta_{\text{H}}\varepsilon_{1}\left(\mu_{M}\gamma_{1}\tau_{1}-J_{1}J_{9}-\beta_{\text{T}}^{*}\varepsilon_{1}s_{0}J_{9}\right),\\ a_{4}=\left(\mu_{M}\beta_{\text{T}}^{*}\left(b+k\right)+\beta_{\text{T}}^{*}\left(s_{0}+\rho v_{\text{T}0}\right)\varepsilon_{1}\beta_{\text{H}}+\beta_{\text{H}}\varepsilon_{1}\left(b+k\right)\right). \end{array}$$

To determine the sign of *b*, we find the subsequent nonvanishing partial derivatives of *F*.

(30) $$\begin{array}{c} \frac{\partial^{2}f_{1}}{\partial x_{4}\partial \beta_{\text{T}}^{*}}=-s_{0},\\ \frac{\partial^{2}f_{1}}{\partial x_{6}\partial \beta_{\text{T}}^{*}}=-\sigma s_{0},\\ \frac{\partial^{2}f_{3}}{\partial x_{4}\partial \beta_{\text{T}}^{*}}=s_{0}+\rho v_{\text{T}0},\\ \frac{\partial^{2}f_{3}}{\partial x_{6}\partial \beta_{\text{T}}^{*}}=\sigma \left(s_{0}+\rho v_{\text{T}0}\right). \end{array}$$

Therefore, *b* = (*β*_T_^∗^*k*(*s*_0_ + *ρv*_T0_)^2^/(*b* + *k*)^2^)*w*_4_*v*_4_.

The article "Modeling the Effects of Helminth Infection on the Transmission Dynamics of Mycobacterium tuberculosis under Optimal Control Strategies" was published in 2020. Journal: Comput Math Methods Med.

Now, according to [25], the signs of *a* and *b* dictate the local dynamics; thus, we have the following lemma.

**Lemma 1 .**

Suppose that *b* > 0. Then, we have the following:

- System (4) undergoes backward bifurcation if the coefficient *a* is positive
- System (4) will exhibit transcritical bifurcation if the coefficient *a* is negative

## 3. Sensitivity Analysis

In this section, we perform a sensitivity analysis of the effective reproduction number subject to each parameter in order to determine the impact of every parameter on the effective reproduction number. Therefore, we compute the forward sensitivity index of the effective reproduction number *ℛ*_HT_ with respect to the parameters using the approach by Chitnis et al. [26]. Since *ℛ*_HT_ = max{*ℛ*_H_, *ℛ*_T_}, then the sensitivity indices for *ℛ*_H_ and *ℛ*_T_ are computed. The normalized forward sensitivity index of a variable *P* with respect to parameter *r* is defined as *ζ*_*r*_^*P*^ = (*r*/*P*)(*∂P*/*∂r*). For instance, the sensitivity index of *ℛ*_T_ with respect to *β*_T_ is given by *ζ*_*β*_T__^*ℛ*_T_^ = (*β*_T_/*ℛ*_T_)(*∂ℛ*_T_/*β*_T_) = 1, and other indices are evaluated using parameter values in Table 1. The remaining indices are given in Tables 2 and 3.

The article "Modeling the Effects of Helminth Infection on the Transmission Dynamics of Mycobacterium tuberculosis under Optimal Control Strategies" was published in 2020. Journal: Comput Math Methods Med.

From Tables 2 and 3, the most positive parameter indices are *β*_T_, *k*, and *β*_H_ while the most negative parameter indices are *b*, *d*_T_, and *μ*_*M*_. This implies that when parameters*β*_T_,*k*, and*β*_H_are increased, and while the remaining are kept constant, the endemicity of the disease is increased, while when the parameter*μ*_*M*_is increased, the endemicity of disease is decreased. Increasing the natural birth rate and Mtb mortality rate does not make biological sense that the disease would be contained. Thus, we suggest the application of optimal control to sensitive parameters such as *β*_H_, *β*_T_, and *μ*_*M*_ to study how effectively we can contain the helminth-Mtb infection.

## 4. The Optimal Control Problem

In this section, the extension of model (1) is formed by including four time-dependent controls so as to decide the optimal strategy for controlling the two diseases. The controls are defined as follows:

- Educational campaign *u*_1_(*t*) that sensitizes the parents to vaccinate more infants. Therefore, the recruitment for the Mtb-vaccinated individuals changes to *ηN*(1 + *u*_1_(*t*)) meaning that when this control is 100% implemented, then the number of vaccinated babies doubles
- Treatment *α*_1_*u*_2_(*t*) of individuals with active TB, where *α*_1_ is the drug efficacy use for Mtb infection. Therefore, the Mtb recovery rate changes to *τ*_2_ + *α*_1_*u*_2_(*t*)
- Deworming at a rate *α*_2_*u*_3_(*t*) for the helminth-infected individuals and coinfected individuals, where *α*_2_ is the drug efficacy use for helminth infection. Therefore, the helminth recovery rate changes to *τ*_1_ + *α*_2_*u*_3_(*t*)
- Sanitation and proper hygiene *u*_4_ that reduces the ingestion rate of parasites. Therefore, the force of infection for the helminth infection is changed to *λ*_H_ = (1 − *u*_4_)*β*_H_*M*/(*K* + *M*)

After incorporating the controls *u*_1_(*t*), *u*_2_(*t*), *u*_3_(*t*), and *u*_4_(*t*) in the Mtb-helminth infection model (4), then the optimal control model becomes

(31) $$\begin{array}{c} \left(\begin{array}{c} \frac{dS}{dt}=\left(1-\eta \right)bN+\gamma_{1}R_{\text{H}}+\gamma_{2}R_{\text{T}}-\left(\mu +\lambda_{\text{T}}+\left(1-u_{4}\right)\lambda_{\text{H}}\right)S,\\ \frac{dV_{\text{T}}}{dt}=\eta b\left(1+u_{1}\right)N-\left(\mu +\rho \lambda_{\text{T}}+\left(1-u_{4}\right)\lambda_{\text{H}}\right)V_{\text{T}},\\ \frac{dE_{\text{T}}}{dt}=\lambda_{\text{T}}S+\rho \lambda_{\text{T}}V_{\text{T}}+\lambda_{\text{T}}R_{\text{H}}-\left(\mu +k+\left(1-u_{4}\right)\lambda_{\text{H}}\right)E_{\text{T}},\\ \frac{dI_{\text{T}}}{dt}=kE_{\text{T}}+\left(\tau_{1}+\alpha_{2}u_{3}\right)I_{\text{HT}}-\left(\mu +d_{\text{T}}+\tau_{2}+\left(1-u_{4}\right)\lambda_{\text{H}}\right)I_{\text{T}}-\left(\tau_{2}+\alpha_{1}u_{2}\right)I_{\text{T}},\\ \frac{dI_{\text{H}}}{dt}=\left(1-u_{4}\right)\lambda_{\text{H}}S+\left(1-u_{4}\right)\lambda_{\text{H}}V_{\text{T}}+\left(1-u_{4}\right)\lambda_{\text{H}}R_{\text{T}}+\tau_{2}I_{\text{HT}}-\left(g\lambda_{\text{T}}+\mu +d_{\text{H}}+\varepsilon_{1}\right)I_{\text{H}}-\left(\tau_{1}+\alpha_{2}u_{3}\right)I_{\text{H}},\\ \frac{dI_{\text{HT}}}{dt}=g\lambda_{\text{T}}I_{\text{H}}+\left(1-u_{4}\right)\lambda_{\text{H}}\left(E_{\text{T}}+I_{\text{T}}\right)-\left(\mu +d_{\text{HT}}+\tau_{2}+\varepsilon_{2}\right)I_{\text{HT}}-\left(\tau_{1}+\alpha_{2}u_{3}\right)I_{\text{HT}},\\ \frac{dR_{\text{T}}}{dt}=\left(\tau_{2}+\alpha_{1}u_{2}\right)I_{\text{T}}-\left(\left(1-u_{4}\right)\lambda_{\text{H}}+\mu +\gamma_{2}\right)R_{\text{T}},\\ \frac{R_{\text{H}}}{dt}=\left(\tau_{1}+\alpha_{2}u_{3}\right)I_{\text{H}}-\left(\lambda_{\text{T}}+\mu +\gamma_{1}\right)R_{\text{H}},\\ \frac{dM}{dt}=\varepsilon_{1}I_{\text{H}}+\varepsilon_{2}I_{\text{HT}}-\mu_{M}M. \end{array}\right. \end{array}$$

We employ Pontryagin's Maximum Principle to figure out the required conditions for the optimal control of helminth-Mtb coinfection. The control set *U* is Lebesgue measurable and is defined as *U* = {*u*_1_(*t*), *u*_2_(*t*), *u*_3_(*t*), *u*_4_(*t*): 0 ≤ *u*_*i*_(*t*) ≤ 1, 0 < *t* ≤ *t*_*f*_}. Then, the objective is to minimize individuals with active TB, individuals infested with helminth parasites, and coinfected individuals while keeping the cost low. For this problem, we consider the objective functional defined by

(32) $$\begin{array}{c} J=\int_{t_{0}}^{t_{f}}\left\{C_{1}I_{\text{T}}+C_{2}I_{\text{H}}+C_{3}I_{\text{HT}}+\frac{1}{2}\overset{4}{\underset{i=1}{\sum }}w_{i}u_{i}^{2}\right\}dt, \end{array}$$

where *C*_1_*I*_T_, *C*_2_*I*_H_, are *C*_3_*I*_HT_ are the costs related to active tuberculosis individuals, individuals infected with helminths, and coinfected individuals, respectively. The expression (1/2)*w*_*i*_*u*_*i*_^2^ is related to the background costs with relative cost weights *w*_*i*_ for every control measure. The quadratic cost is tailored as utilized in other models with controls (see [16, 27]). The particular value of the weights requires intensive data processing; hence, we elect estimate values for theoretical purposes.

The article "Modeling the Effects of Helminth Infection on the Transmission Dynamics of Mycobacterium tuberculosis under Optimal Control Strategies" was published in 2020. Journal: Comput Math Methods Med.

The aim is to minimize the objective functional *J* as defined in (32) subject to model (31). Therefore, we seek to get the optimal controls *u*_1_^∗^, *u*_2_^∗^, *u*_3_^∗^, and *u*_4_^∗^ such that

(33) $$\begin{array}{c} J\left(u_{1}^{*},u_{2}^{*},u_{3}^{*},u_{4}^{*}\right)=\underset{u_{1},u_{2},u_{3},u_{4}\in U}{\min}J\left(u_{1},u_{2},u_{3},u_{4}\right), \end{array}$$

where *U* = {(*u*_1_, *u*_2_, *u*_3_, *u*_4_)andthereforethecontrolss*u*_1_, *u*_2_, *u*_3_, are*u*_4_aremeasurablewith0 ≤ *u*_1_ ≤ 1, 0 ≤ *u*_2_ ≤ 1, 0 ≤ *u*_3_ ≤ 1, and0 ≤ *u*_4_ ≤ 1for*t* ∈ [*t*_0_*t*_*f*_]}.

**Theorem 3 .**

Consider the control problem with the system of equations in (31). There exist *u*^∗^ = (*u*_1_^∗^, *u*_2_^∗^, *u*_3_^∗^, *u*_4_^∗^) ∈ *U* such that

(34) $$\begin{array}{c} \underset{u_{1},u_{2},u_{3},u_{4}\in U}{\min}J\left(u_{1},u_{2},u_{3},u_{4},\right)=J\left(u_{1}^{*},u_{2}^{*},u_{3}^{*},u_{4}^{*}\right). \end{array}$$

The necessary conditions that an optimal solution must satisfy are derived from Pontryagin's Maximum Principle [28]. The principle converts equations (31) and (32) into the problem of minimizing the pointwise Hamiltonian *H*, with reference to *u*_1_, *u*_2_, *u*_3_, and *u*_4_. The Hamiltonian is given by

(35) $$\begin{array}{c} H=C_{1}I_{\text{T}}+C_{2}I_{\text{H}}+C_{3}I_{\text{HT}}+\frac{1}{2}\left(w_{1}u_{1}^{2}+w_{2}u_{2}^{2}+w_{3}u_{3}^{2}+w_{4}u_{4}^{2}\right)+\lambda_{S}\left\{\left(1-\eta \right)bN+\gamma_{1}R_{\text{H}}+\gamma_{2}R_{\text{T}}-\left(\mu +\lambda_{\text{T}}+\left(1-u_{4}\right)\lambda_{\text{H}}\right)S\right\}+\lambda_{V_{\text{T}}}\left\{\eta b\left(1+u_{1}\right)N-\left(\mu +\rho \lambda_{\text{T}}+\left(1-u_{4}\right)\lambda_{\text{H}}\right)V_{\text{T}}\right\}+\lambda_{E_{\text{T}}}\left\{\lambda_{\text{T}}S\right.+\rho \lambda_{\text{T}}V_{\text{T}}+\lambda_{\text{T}}R_{\text{H}}-\left(\mu +k+\left(1-u_{4}\right)\lambda_{\text{H}}\right)E_{\text{T}}+\lambda_{I_{\text{T}}}\left\{kE_{\text{T}}+\left(\tau_{1}+\alpha_{2}u_{3}\right)I_{\text{HT}}-\left(\mu +d_{\text{T}}+\left(1-u_{4}\right)\lambda_{\text{H}}\right)I_{\text{T}}-\left(\tau_{2}+\alpha_{1}u_{2}\right)I_{\text{T}}\right\}+\lambda_{I_{\text{H}}}\left\{\left(1-u_{4}\right)\lambda_{\text{H}}\left(S+V_{\text{T}}+R_{\text{T}}\right)+\tau_{2}I_{\text{HT}}-\left(\mu +d_{\text{H}}+\varepsilon_{1}+g\lambda_{\text{T}}\right)I_{\text{H}}-\left(\tau_{1}+\alpha_{2}u_{3}\right)I_{\text{H}}\right\}+\lambda_{I_{\text{HT}}}\left\{g\lambda_{\text{T}}I_{\text{H}}+\left(1-u_{4}\right)\lambda_{\text{H}}\left(E_{\text{T}}+I_{\text{T}}\right)-\left(\mu +d_{\text{HT}}+\tau_{2}+\varepsilon_{2}\right)I_{\text{HT}}-\left(\tau_{1}+\alpha_{2}u_{3}\right)I_{\text{HT}}\right\}+\lambda_{R_{\text{T}}}\left\{\left(\tau_{2}+\alpha_{1}u_{2}\right)I_{\text{T}}-\left(\lambda_{\text{H}}+\mu +\gamma_{2}\right)R_{\text{T}}\right\}+\lambda_{R_{\text{H}}}\left\{\left(\tau_{1}+\alpha_{2}u_{3}\right)I_{\text{H}}-\left(\lambda_{\text{T}}+\mu +\gamma_{1}\right)R_{\text{H}}\right\}+\lambda_{M}\left\{\varepsilon_{1}I_{\text{H}}+\varepsilon_{2}I_{\text{HT}}-\mu_{M}M\right\}. \end{array}$$

where *λ*_*S*_, *λ*_*V*_T__, *λ*_*E*_T__, *λ*_*I*_T__, *λ*_*I*_H__, *λ*_*I*_HT__, *λ*_*R*_T__, *λ*_*R*_H__, and *λ*_*M*_ are the costate variables or the adjoint variables. Now, applying Pontryagin's Maximum Principle [28], the problem has a solution following the results of the optimal control problem in [29].

The article "Modeling the Effects of Helminth Infection on the Transmission Dynamics of Mycobacterium tuberculosis under Optimal Control Strategies" was published in 2020. Journal: Comput Math Methods Med.

**Theorem 4 .**

Given the optimal control*u*_*i*_, for*i* = 1, 2, 3, 4, and the solutions*S*,*V*_T_,*E*_T_,*I*_T_,*I*_H_,*I*_HT_,*R*_T_,*R*_H_, and*M*, and the state systems (31) and (32) that minimize*J*(*u*_1_, *u*_2_, *u*_3_, *u*_4_)over*U*, there exist adjoint variables*λ*_*S*_,*λ*_*V*_T__,*λ*_*E*_T__,*λ*_*I*_T__,*λ*_*I*_H__,*λ*_*I*_HT__,*λ*_*R*_T__,*λ*_*R*_H__, and*λ*_*M*_ satisfying

(36) $$\begin{array}{c} -\frac{d\lambda_{i}}{dt}=\frac{\partial H}{\partial x_{i}} \end{array}$$

where *x*_*i*_ = *S*, *V*_T_, *I*_T_, *I*_H_, *I*_HT_, *R*_T_, *R*_H_, *M* with transversality conditions *λ*_*S*_(*t*_*f*_) = *λ*_*V*_T__(*t*_*f*_) = *λ*_*E*_T__(*t*_*f*_) = *λ*_*I*_T__(*t*_*f*_) = *λ*_*I*_H__(*t*_*f*_) = *λ*_*I*_HT__(*t*_*f*_) = *λ*_*R*_T__(*t*_*f*_) = *λ*_*R*_H__(*t*_*f*_) = *λ*_*M*_(*t*_*f*_) = 0, and the subsequent characterization holds on the interior of the control set *U*:

(37) $$\begin{array}{c} u_{1}^{*}=\max\left\{0,\min\left\{1,-\frac{\eta bN\lambda_{V_{\text{T}}}}{w_{1}}\right\}\right\},\\ u_{2}^{*}=\max\left\{0,\min\left\{1,\frac{\alpha_{1}I_{\text{T}}\left(\lambda_{I_{\text{T}}}-\lambda_{R_{\text{T}}}\right)}{w_{2}}\right\}\right\},\\ u_{3}^{*}=\max\left\{0,\min\left\{1,\frac{\alpha_{2}I_{\text{H}}\left(\lambda_{I_{\text{H}}}-\lambda_{R_{\text{H}}}\right)+\alpha_{2}I_{\text{HT}}\left(\lambda_{I_{\text{HT}}}-\lambda_{I_{\text{T}}}\right)}{w_{3}}\right\}\right\},\\ u_{4}^{*}=\max\left\{0,\min\left\{1,\frac{\lambda_{\text{H}}\lambda_{I_{\text{H}}}\left(S+V_{\text{T}}+R_{\text{T}}\right)+\lambda_{\text{H}}\lambda_{I_{\text{HT}}}\left(E_{\text{T}}+I_{\text{T}}\right)}{w_{4}}-\frac{\lambda_{\text{H}}\left(S\lambda_{S}+V_{\text{T}}\lambda_{V_{\text{T}}}+E_{\text{T}}\lambda_{E_{\text{T}}}+I_{\text{T}}\lambda_{I_{\text{T}}}\right)}{w_{4}}\right\}\right\}. \end{array}$$

**Proof**

Flemming and Rishel [23] provide the existence of an optimal control model (31) and the costate variables (36) due to the boundness of state equations and the Lipschitz structure of the ordinary differential equations. Therefore, applying the necessary conditions from Pontryagin's Maximum Principle, we obtain the following system for costate variables:

(38) $$\begin{array}{c} \frac{d\lambda_{S}}{dt}=-\left(1-\eta \right)b\lambda_{S}+\frac{\beta_{\text{T}}\left(I_{\text{T}}+\sigma I_{\text{HT}}\right)S}{N^{2}}\left(\lambda_{E_{\text{T}}}-\lambda_{S}\right)+\frac{\beta_{\text{T}}\left(I_{\text{T}}+\sigma I_{\text{HT}}\right)V_{\text{T}}}{N^{2}}\left(\rho \lambda_{E_{\text{T}}}-\lambda_{V_{\text{T}}}\right)-\eta b\left(1+u_{1}\right)\lambda_{V_{\text{T}}}+\frac{\beta_{\text{T}}\left(I_{\text{T}}+\sigma I_{\text{HT}}\right)R_{\text{H}}}{N^{2}}\left(\lambda_{E_{\text{T}}}-\lambda_{R_{\text{H}}}\right)+\frac{\beta_{\text{T}}\left(I_{\text{T}}+\sigma I_{\text{HT}}\right)}{N}\left(\lambda_{S}-\lambda_{E_{\text{T}}}\right)+\frac{g\beta_{\text{T}}\left(I_{\text{T}}+\sigma I_{\text{HT}}\right)I_{\text{H}}}{N^{2}}\left(\lambda_{I_{\text{HT}}}-\lambda_{I_{\text{H}}}\right)+\frac{\left(1-u_{4}\right)\beta_{\text{H}}M}{K+M}\left(\lambda_{S}-\lambda_{I_{\text{H}}}\right)+\mu \lambda_{S},\\ \frac{d\lambda_{V_{\text{T}}}}{dt}=-\left(1-\eta \right)b\lambda_{S}+\frac{\beta_{\text{T}}\left(I_{\text{T}}+\sigma I_{\text{HT}}\right)V_{\text{T}}}{N^{2}}\left(\rho \lambda_{E_{\text{T}}}-\lambda_{V_{\text{T}}}\right)+\frac{\beta_{\text{T}}\left(I_{\text{T}}+\sigma I_{\text{HT}}\right)R_{\text{H}}}{N^{2}}\left(\lambda_{E_{\text{T}}}-\lambda_{R_{\text{T}}}\right)-\eta b\left(1+u_{1}\right)\lambda_{V_{\text{T}}}+\frac{\beta_{\text{T}}\left(I_{\text{T}}+\sigma I_{\text{HT}}\right)S}{N^{2}}\left(\lambda_{E_{\text{T}}}-\lambda_{S}\right)+\frac{\beta_{\text{T}}\left(I_{\text{T}}+\sigma I_{\text{HT}}\right)}{N}\left(\lambda_{V_{\text{T}}}-\rho \lambda_{E_{\text{T}}}\right)+\frac{g\beta_{\text{T}}\left(I_{\text{T}}+\sigma I_{\text{HT}}\right)I_{\text{H}}}{N^{2}}\left(\lambda_{I_{\text{HT}}}-\lambda_{I_{\text{H}}}\right)+\frac{\left(1-u_{4}\right)\beta_{\text{H}}M}{K+M}\left(\lambda_{V_{\text{T}}}-\lambda_{I_{\text{H}}}\right)+\mu \lambda_{V_{\text{T}}},\\ \frac{d\lambda_{E_{\text{T}}}}{dt}=-\left(1-\eta \right)b\lambda_{S}+\frac{\beta_{\text{T}}\left(I_{\text{T}}+\sigma I_{\text{HT}}\right)S}{N^{2}}\left(\lambda_{E_{\text{T}}}-\lambda_{S}\right)+\frac{\rho \beta_{\text{T}}\left(I_{\text{T}}+\sigma I_{\text{HT}}\right)V_{\text{T}}}{N^{2}}\left(\lambda_{E_{\text{T}}}-\lambda_{V_{\text{T}}}\right)-\eta b\left(1+u_{1}\right)\lambda_{V_{\text{T}}}+\frac{\beta_{\text{T}}\left(I_{\text{T}}+\sigma I_{\text{HT}}\right)R_{\text{H}}}{N^{2}}\left(\lambda_{E_{\text{T}}}-\lambda_{R_{\text{H}}}\right)+\frac{g\beta_{\text{T}}\left(I_{\text{T}}+\sigma I_{\text{HT}}\right)I_{\text{H}}}{N^{2}}\left(\lambda_{I_{\text{HT}}}-\lambda_{I_{\text{H}}}\right)+\frac{\left(1-u_{4}\right)\beta_{\text{H}}M}{K+M}\left(\lambda_{E_{\text{T}}}-\lambda_{I_{\text{HT}}}\right)+k\left(\lambda_{E_{\text{T}}}-\lambda_{I_{\text{T}}}\right)+\mu \lambda_{E_{\text{T}}},\\ \frac{d\lambda_{I_{\text{T}}}}{dt}=-C_{1}-\left(1-\eta \right)b\lambda_{S}+\frac{\beta_{\text{T}}\left(I_{\text{T}}+\sigma I_{\text{HT}}\right)S}{N^{2}}\left(\lambda_{E_{\text{T}}}-\lambda_{S}\right)+\frac{\rho \beta_{\text{T}}\left(I_{\text{T}}+\sigma I_{\text{HT}}\right)V_{\text{T}}}{N^{2}}\left(\lambda_{E_{\text{T}}}-\lambda_{V_{\text{T}}}\right)-\eta b\left(1+u_{1}\right)\lambda_{V_{\text{T}}}+\frac{\beta_{\text{T}}\left(I_{\text{T}}+\sigma I_{\text{HT}}\right)R_{\text{H}}}{N^{2}}\left(\lambda_{E_{\text{T}}}-\lambda_{R_{\text{H}}}\right)+\frac{\beta_{\text{T}}\left(S\lambda_{\text{S}}+V_{\text{T}}\lambda_{V_{\text{T}}}+I_{\text{T}}\lambda_{R_{\text{H}}}\right)}{N}+\frac{g\beta_{\text{T}}\left(I_{\text{T}}+\sigma I_{\text{HT}}\right)I_{\text{H}}}{N^{2}}\left(\lambda_{I_{\text{HT}}}-\lambda_{I_{\text{H}}}\right)+\frac{\left(1-u_{4}\right)\beta_{\text{H}}M}{K+M}\left(\lambda_{I_{\text{T}}}-\lambda_{I_{\text{HT}}}\right)+\left(\mu +d_{\text{T}}\right)\lambda_{I_{\text{T}}}+\frac{g\beta_{\text{T}}I_{\text{H}}}{N}\left(\lambda_{I_{\text{H}}}-\lambda_{I_{\text{HT}}}\right)+\left(\tau_{2}+\alpha_{1}u_{2}\right)\left(\lambda_{I_{\text{T}}}-\lambda_{R_{\text{H}}}\right),\\ \frac{d\lambda_{I_{\text{H}}}}{dt}=-C_{2}-\left(1-\eta \right)b\lambda_{S}+\frac{\beta_{\text{T}}\left(I_{\text{T}}+\sigma I_{\text{HT}}\right)S}{N^{2}}\left(\lambda_{E_{\text{T}}}-\lambda_{S}\right)+\frac{\rho \beta_{\text{T}}\left(I_{\text{T}}+\sigma I_{\text{HT}}\right)V_{\text{T}}}{N^{2}}\left(\lambda_{E_{\text{T}}}-\lambda_{V_{\text{T}}}\right)-\eta b\left(1+u_{1}\right)\lambda_{V_{\text{T}}}+\frac{\beta_{\text{T}}\left(I_{\text{T}}+\sigma I_{\text{HT}}\right)R_{\text{H}}}{N^{2}}\left(\lambda_{E_{\text{T}}}-\lambda_{R_{\text{H}}}\right)+\frac{g\beta_{\text{T}}\left(I_{\text{T}}+\sigma I_{\text{HT}}\right)}{N}\left(\lambda_{I_{\text{H}}}-\lambda_{I_{\text{HT}}}\right)+\frac{g\beta_{\text{T}}\left(I_{\text{T}}+\sigma I_{\text{HT}}\right)I_{\text{H}}}{N^{2}}\left(\lambda_{I_{\text{HT}}}-\lambda_{I_{\text{H}}}\right)+\left(\tau_{1}+\alpha_{2}u_{3}\right)\left(\lambda_{I_{\text{H}}}-\lambda_{R_{\text{H}}}\right)+\left(\mu +d_{\text{H}}+\varepsilon_{1}\right)\lambda_{I_{\text{H}}}+\varepsilon_{1}\lambda_{M},\\ \frac{d\lambda_{I_{\text{HT}}}}{dt}=-C_{3}-\left(1-\eta \right)b\lambda_{S}+\frac{\beta_{\text{T}}\left(I_{\text{T}}+\sigma I_{\text{HT}}\right)S}{N^{2}}\left(\lambda_{E_{\text{T}}}-\lambda_{S}\right)+\frac{\rho \beta_{\text{T}}\left(I_{\text{T}}+\sigma I_{\text{HT}}\right)V_{\text{T}}}{N^{2}}\left(\lambda_{E_{\text{T}}}-\lambda_{V_{\text{T}}}\right)-\eta b\left(1+u_{1}\right)\lambda_{V_{\text{T}}}+\frac{\beta_{\text{T}}\left(I_{\text{T}}+\sigma I_{\text{HT}}\right)R_{\text{H}}}{N^{2}}\left(\lambda_{E_{\text{T}}}-\lambda_{R_{\text{H}}}\right)+\frac{\sigma g\beta_{\text{T}}\left(I_{\text{T}}+\sigma I_{\text{HT}}\right)}{N}\left(\lambda_{I_{\text{H}}}-\lambda_{I_{\text{HT}}}\right)+\frac{g\beta_{\text{T}}\left(I_{\text{T}}+\sigma I_{\text{HT}}\right)I_{\text{H}}}{N^{2}}\left(\lambda_{I_{\text{HT}}}-\lambda_{I_{\text{H}}}\right)+\left(\tau_{1}+\alpha_{2}u_{3}\right)\left(\lambda_{I_{\text{HT}}}-\lambda_{I_{\text{T}}}\right)+\left(\mu +d_{\text{HT}}+\tau_{2}+\varepsilon_{2}\right)\lambda_{I_{\text{HT}}}+\varepsilon_{2}\lambda_{M}-\tau_{2}\lambda_{I_{\text{H}}}+\frac{\beta_{T}\sigma \left(S\lambda_{S}+\rho V_{\text{T}}\lambda_{V_{\text{T}}}+R_{\text{H}}\lambda_{R_{\text{H}}}\right)}{N}-\frac{\sigma \beta_{\text{T}}\left(S+\rho V_{\text{T}}+R_{\text{H}}\right)}{N},\\ \frac{d\lambda_{R_{\text{T}}}}{dt}=-\left(1-\eta \right)b\lambda_{S}+\frac{\beta_{\text{T}}\left(I_{\text{T}}+\sigma I_{\text{HT}}\right)S}{N^{2}}\left(\lambda_{E_{\text{T}}}-\lambda_{S}\right)+\frac{\rho \beta_{\text{T}}\left(I_{\text{T}}+\sigma I_{\text{HT}}\right)V_{\text{T}}}{N^{2}}\left(\lambda_{E_{\text{T}}}-\lambda_{V_{\text{T}}}\right)-\eta b\left(1+u_{1}\right)\lambda_{V_{\text{T}}}+\frac{\beta_{\text{T}}\left(I_{\text{T}}+\sigma I_{\text{HT}}\right)R_{\text{H}}}{N^{2}}\left(\lambda_{E_{\text{T}}}-\lambda_{R_{\text{H}}}\right)+\gamma_{2}\left(\lambda_{R_{\text{T}}}-\lambda_{S}\right)+\mu \lambda_{R_{\text{T}}}+\frac{g\beta_{\text{T}}\left(I_{\text{T}}+\sigma I_{\text{HT}}\right)I_{\text{H}}}{N^{2}}\left(\lambda_{I_{\text{HT}}}-\lambda_{I_{\text{H}}}\right)+\frac{\left(1-u_{4}\right)\beta_{\text{H}}M}{K+M}\left(\lambda_{\lambda_{R_{\text{T}}}}-\lambda_{I_{\text{H}}}\right),\\ \frac{d\lambda_{R_{\text{T}}}}{dt}=-\left(1-\eta \right)b\lambda_{S}+\frac{\beta_{\text{T}}\left(I_{\text{T}}+\sigma I_{\text{HT}}\right)S}{N^{2}}\left(\lambda_{E_{\text{T}}}-\lambda_{S}\right)+\frac{\rho \beta_{\text{T}}\left(I_{\text{T}}+\sigma I_{\text{HT}}\right)V_{\text{T}}}{N^{2}}\left(\lambda_{E_{\text{T}}}-\lambda_{V_{\text{T}}}\right)-\eta b\left(1+u_{1}\right)\lambda_{V_{\text{T}}}+\frac{\beta_{\text{T}}\left(I_{\text{T}}+\sigma I_{\text{HT}}\right)R_{\text{H}}}{N^{2}}\left(\lambda_{E_{\text{T}}}-\lambda_{R_{\text{H}}}\right)+\gamma_{1}\left(\lambda_{R_{\text{H}}}-\lambda_{S}\right)+\mu \lambda_{R_{\text{H}}}+\frac{g\beta_{\text{T}}\left(I_{\text{T}}+\sigma I_{\text{HT}}\right)I_{\text{H}}}{N^{2}}\left(\lambda_{I_{\text{HT}}}-\lambda_{I_{\text{H}}}\right)+\frac{\beta_{\text{T}}\left(I_{\text{T}}+\sigma I_{\text{HT}}\right)}{N}\left(\lambda_{\lambda_{R_{\text{H}}}}-\lambda_{E_{\text{T}}}\right),\\ \frac{d\lambda_{M}}{dt}=\frac{\left(1-u_{4}\right)\beta_{\text{H}}MS}{{\left(K+M\right)}^{2}}\left(\lambda_{I_{\text{H}}}-\lambda_{S}\right)+\frac{\left(1-u_{4}\right)\beta_{\text{H}}MV_{\text{T}}}{{\left(K+M\right)}^{2}}\left(\lambda_{I_{\text{H}}}-\lambda_{V_{\text{T}}}\right)+\frac{\left(1-u_{4}\right)\beta_{\text{H}}MR_{\text{T}}}{{\left(K+M\right)}^{2}}\left(\lambda_{I_{\text{H}}}-\lambda_{R_{\text{T}}}\right)+\frac{\left(1-u_{4}\right)\beta_{\text{H}}ME_{\text{T}}}{{\left(K+M\right)}^{2}}\left(\lambda_{I_{\text{HT}}}-\lambda_{E_{\text{T}}}\right)+\frac{\left(1-u_{4}\right)\beta_{\text{H}}MI_{\text{T}}}{{\left(K+M\right)}^{2}}\left(\lambda_{I_{\text{HT}}}-\lambda_{I_{\text{T}}}\right)+\frac{\left(1-u_{4}\right)\beta_{\text{H}}\left(S\lambda_{S}+V_{\text{T}}\lambda_{V_{\text{T}}}+E_{\text{T}}\lambda_{E_{\text{T}}}+I_{\text{T}}\lambda_{I_{\text{T}}}+R_{\text{T}}\lambda_{R_{\text{T}}}\right)}{K+M}+\mu_{M}\lambda_{M}-\frac{\left(1-u_{4}\right)\beta_{\text{H}}\left(\left(S+V_{\text{T}}+R_{\text{T}}\right)\lambda_{I_{\text{H}}}+\left(E_{\text{T}}+I_{\text{T}}\right)\lambda_{I_{\text{HT}}}\right)}{K+M}. \end{array}$$

To get the controls, we solve the equations *∂H*/*∂u*_*i*_ = 0 at *u*_*i*_^∗^ for *i* = 1, ⋯, 4 and obtained the following:

(39) $$\begin{array}{c} u_{1}^{*}=-\frac{\eta bN\lambda_{V_{\text{T}}}}{w_{1}},\\ u_{2}^{*}=\frac{\alpha_{1}I_{\text{T}}\left(\lambda_{I_{\text{T}}}-\lambda_{R_{\text{T}}}\right)}{w_{2}},\\ u_{3}^{*}=\frac{\alpha_{2}I_{\text{H}}\left(\lambda_{I_{\text{H}}}-\lambda_{R_{\text{H}}}\right)+\alpha_{2}I_{\text{HT}}\left(\lambda_{I_{\text{HT}}}-\lambda_{I_{\text{T}}}\right)}{w_{4}},\\ u_{4}^{*}=\frac{\lambda_{\text{H}}\lambda_{I_{\text{H}}}\left(S+V_{\text{T}}+R_{\text{T}}\right)+\lambda_{\text{H}}\lambda_{I_{\text{HT}}}\left(E_{\text{T}}+I_{\text{T}}\right)}{w_{4}}-\lambda_{\text{H}}\left(S\lambda_{S}+V_{\text{T}}\lambda_{V_{\text{T}}}+E_{\text{T}}\lambda_{E_{\text{T}}}+I_{\text{T}}\lambda_{I_{\text{T}}}\right). \end{array}$$

Then, we write by standard control arguments involving the bounds on the controls as

(40) $$\begin{array}{c} \begin{array}{c} u_{1}^{*}=\left(\begin{array}{c} \Theta_{1},\text{if}0<\Theta_{1}<1,\\ 0,\text{if}\Theta_{1}\leq 0,\\ 1,\text{if}\Theta_{1}\geq 1, \end{array}\right. \end{array}\\ \begin{array}{c} u_{2}^{*}=\left(\begin{array}{c} \Theta_{2},\text{if}0<\Theta_{2}<1,\\ 0,\text{if}\Theta_{2}\leq 0,\\ 1,\text{if}\Theta_{2}\geq 1, \end{array}\right. \end{array}\\ \begin{array}{c} u_{3}^{*}=\left(\begin{array}{c} \Theta_{3},\text{if}0<\Theta_{3}<1,\\ 0,\text{if}\Theta_{3}\leq 0,\\ 1,\text{if}\Theta_{3}\geq 1, \end{array}\right. \end{array}\\ \begin{array}{c} u_{4}^{*}=\left(\begin{array}{c} \Theta_{4},\text{if}0<\Theta_{4}<1,\\ 0,\text{if}\Theta_{4}\leq 0,\\ 1,\text{if}\Theta_{4}\geq 1, \end{array}\right. \end{array} \end{array}$$

where

(41) $$\begin{array}{c} \Theta_{1}=-\frac{\eta bN\lambda_{V_{\text{T}}}}{w_{1}},\\ \Theta_{2}=\frac{\alpha_{1}I_{\text{T}}\left(\lambda_{I_{\text{T}}}-\lambda_{R_{\text{T}}}\right)}{w_{2}},\\ \Theta_{3}=\frac{\alpha_{2}I_{\text{H}}\left(\lambda_{I_{\text{H}}}-\lambda_{R_{\text{H}}}\right)+\alpha_{2}I_{\text{HT}}\left(\lambda_{I_{\text{HT}}}-\lambda_{I_{\text{T}}}\right)}{w_{4}},\\ \Theta_{4}=\frac{\lambda_{\text{H}}\lambda_{I_{\text{H}}}\left(S+V_{\text{T}}+R_{\text{T}}\right)+\lambda_{\text{H}}\lambda_{I_{\text{HT}}}\left(E_{\text{T}}+I_{\text{T}}\right)}{w_{4}}-\lambda_{\text{H}}\left(S\lambda_{S}+V_{\text{T}}\lambda_{V_{\text{T}}}+E_{\text{T}}\lambda_{E_{\text{T}}}+I_{\text{T}}\lambda_{I_{\text{T}}}\right). \end{array}$$

The article "Modeling the Effects of Helminth Infection on the Transmission Dynamics of Mycobacterium tuberculosis under Optimal Control Strategies" was published in 2020. Journal: Comput Math Methods Med.

## 5. Numerical Simulation

In this section, different optimal control strategies are used to investigate numerically their effect on the spread of helminth and Mtb coinfection. The state system (31), the adjoint system (38), and therefore the characterization in equation (37) are solved numerically using an iterative scheme so as to attain the optimal control. Using the initial conditions for the state system and the transversality conditions for the adjoint system with the initial guess of the controls, we solve the state system forward in time and the adjoint system backward in time using the fourth-order Runge-Kutta scheme with the current solutions of the state system. Then, the controls are updated using a convex combination of the controls and the values from characterization (37). The solution of the state system and the adjoint system is repeated until the present iteration is close to the previous iteration [30].

In numerical simulation, the weights are assumed to depend on the cost of investment and importance of the controls. For example, the cost associated with control *u*_2_ requires huge investment that includes clinical examination of Mtb cases and procurement and transportation of the drugs. The cost associated with control *u*_2_ requires procurement and transportation of antihelminthic drugs and monitoring of the distribution of drugs. We choose the weights as *C*_1_ = 5822, *C*_2_ = 0.89, *C*_3_ = 5822.89, *w*_1_ = 20, *w*_2_ = 40, *w*_3_ = 30, and *w*_4_ = 10 and the initial state variables as *S* = 1500, *V*_T_ = 2000, *E*_T_ = 200, *I*_T_ = 150, *I*_H_ = 100, *I*_HT_ = 80, *R*_T_ = 5, *R*_H_ = 5, and *M* = 200. The efficacy parameters are *α*_1_ = 0.75 and *α*_2_ = 0.8, and the remaining parameter values are given in Table 1.

### 5.1. Control with Educational Campaign (*u*_1_) and Treatment of Individuals with Active TB (*u*_2_)

The educational campaign control (*u*_1_) and treatment of individuals with active TB control (*u*_2_) are used to optimize the objective functional *J* while the other controls (*u*_3_) and (*u*_4_) related to helminths were set to zero. We observed that in Figure 2(b) the number of individuals with active TB was controlled but starts to increase again until the end of the intervention period. This may be related to our previous analysis that helminth infection enhances Mtb infection. In this strategy, helminth infection is not controlled; Figures 2(c) and 2(d) indicate that there is slight significance in the case with controls and without controls for helminth-infected individuals and coinfected individuals, respectively.  Figure 2(e) indicates that the parasite population is not controlled with this strategy while Figure 2(f) indicates that the educational campaign control should be seized after 158 days while treatment of individuals with active TB control should be kept maximum in the entire period of intervention.

The article "Modeling the Effects of Helminth Infection on the Transmission Dynamics of Mycobacterium tuberculosis under Optimal Control Strategies" was published in 2020. Journal: Comput Math Methods Med.

### 5.2. Control with Mass Drug Administration (*u*_3_) and Sanitation (*u*_4_)

The mass drug administration (MDA) control (*u*_3_) and sanitation control (*u*_4_) were used to optimize the objective functional *J*. Again, we observe that Figure 3(a) indicates the increase in vaccinated individuals. Also, Figure 3(b) indicates that the number of people with active TB increases rapidly and is eventually controlled after 55 days. An equivalent scenario is observed in Figures 3(c) and 3(d) where the helminth-infected individuals and coinfected individuals were effectively controlled.  Figure 3(e) suggests that the parasite population is substantially controlled at the end of the intervention period. This strategy seems to be effective in controlling the two diseases from the community.  Figure 3(f) indicates that MDA and sanitation controls should be kept maximum throughout the intervention period.

### 5.3. Control with Educational Campaign (*u*_1_) and Sanitation (*u*_4_)

The educational campaign control (*u*_1_) and sanitation control (*u*_4_) are employed to optimize the objective functional *J*. This strategy has the same profiles as the strategy with mass drug administration and sanitation controls but takes a long time to control the two diseases.  Figure 4(f) indicates that the educational campaign must be stopped after 30 days whereas sanitation control must be kept maximum in the entire period of intervention.

### 5.4. Control with Treatment of Individuals with Active TB (*u*_2_) and MDA (*u*_3_)

The treatment of individuals with active TB control (*u*_2_) and MDA control (*u*_3_) are used to optimize the objective functional *J* while the other controls (*u*_1_) and (*u*_4_) are set to zero.  Figure 5(a) indicates a slight increase in vaccinated individuals compared to the other strategies (Sections 5.1, 5.2, and 5.3). Figures 5(b) and 5(d) indicate that the treatment of individuals with active TB and coinfected individuals is effectively controlled while Figure 5(c) indicates a decrease in the helminth-infected individuals but a rise at the final intervention period. This is due to the absence of preventive measures in this strategy.  Figure 5(f) indicates that both controls should be kept maximum until the final intervention period.

The article "Modeling the Effects of Helminth Infection on the Transmission Dynamics of Mycobacterium tuberculosis under Optimal Control Strategies" was published in 2020. Journal: Comput Math Methods Med.

### 5.5. Control with Educational Campaign (*u*_1_), Treatment of Mtb-Infected Individuals (*u*_2_), MDA (*u*_3_), and Sanitation (*u*_4_)

With this strategy, all four controls are employed to optimize the objective functional *J*. We observed that Figure 6(a) indicates that the number of vaccinated individuals increases more at the end of the intervention period. Figures 6(b)–6(d) indicate that individuals with active TB, helminth-infected individuals, and coinfected individuals are all effectively and efficiently controlled at the end of the intervention period.  Figure 6(e) depicts that the parasite population is decreased to a number that cannot harm the human population. This strategy indicates that optimal educational campaign, treatment of individuals with active TB, MDA, and sanitation would effectively control the helminth-Mtb infection at the end of the intervention period.  Figure 6(f) suggests that the educational campaign should be stopped after 115 days whereas the remaining controls should be maintained maximum for the whole intervention period.

## 6. Discussions and Conclusions

In this paper, we described and formulated a deterministic model for the transmission dynamics and control of helminth-Mtb coinfection. The effective reproduction number was computed, and we explored the steadiness of the disease-free equilibrium point. We again established the existence of backward or forward bifurcation using the Center Manifold Theorem. Then, we investigated the impact the two diseases have on each other and found that helminth infection cases increase Mtb infection cases. In Section 4, we modified the helminth-Mtb model by incorporating four control measures: educational campaign to sensitize the parents to take babies to the BCG vaccine clinic, treatment of individuals with active TB, mass drug administration for helminth and coinfected individuals, and sanitation to reduce the intake rate of parasites. The optimal control was analyzed using Pontryagin's Maximum Principle [28], by first finding the Hamiltonian, the costate variables, the characterization of the controls, and the optimality system.

The article "Modeling the Effects of Helminth Infection on the Transmission Dynamics of Mycobacterium tuberculosis under Optimal Control Strategies" was published in 2020. Journal: Comput Math Methods Med.

Then, we solved numerically the optimality system by the iterative scheme using the Forward-Backward Sweep Method (FBSM) with the combination of the following control measures:

- By applying a combination of educational campaign and treatment of individuals with active TB
- By applying a combination of mass drug administration (MDA) and sanitation
- By applying a combination of educational campaign and sanitation
- By applying a combination of treatment of individuals with active TB and mass drug administration
- By applying a combination of educational campaign, treatment of individuals with active TB, mass drug administration, and sanitation

The control strategies which focus on TB only while helminths are not controlled would not lead to the efficient and effective control of TB or helminth infection. Moreover, control strategies that focus on helminths only while TB is not controlled would control both TB and helminth infections. This is linked to the increased susceptibility of Mtb for individuals infested with helminths. However, control strategies that include all control measures would effectively control the helminth-Mtb coinfection at the end of the intervention period. Thus, we suggest to the public health stakeholders that in order to control the helminth-Mtb coinfection, the intervention strategies that target controlling helminth infection and vaccination of babies with BCG after birth and treatment of individuals with active tuberculosis should be emphasized. One of the limitations of this study is the number of compartments involved that hinders some analytical analyses; however, numerical simulation shows the convergence.

## Figures and Tables

**Figure 1:** Compartmental diagram for the helminth and Mycobacterium tuberculosis coinfection. The dotted lines indicate the interaction of individuals with the polluted environment.

**Figure 2:** Simulations of the helminth-Mtb coinfection model with the effect of educational campaign and treatment of Mtb-infected individuals.

**Figure 3:** Simulations of the helminth-Mtb coinfection model with the effect of MDA and sanitation.

**Figure 4:** Simulations of the helminth-Mtb coinfection model with the effect of educational campaign and sanitation.

**Figure 5:** Simulations of the helminth-Mtb coinfection model with the effect of treatment of Mtb-infected individuals and MDA.

**Figure 6:** Simulations of the helminth-Mtb coinfection model with the effect of educational campaign, treatment of Mtb-infected individuals, MDA, and sanitation.

**Table 1:** Description of the model parameters.

Parameters	Definition	Estimated value	Reference
*b*	Natural birth rate	1/18250day^−1^	[14]
*β*_T_	Transmission rate for Mtb	0.42day^−1^	[15]
*μ*	Natural death rate	1/(60 × 365)day^−1^	[16]
*γ*_1_	Loss of temporary immunity for helminth-recovered individuals	1/70day^−1^	
			Assumed
*β*_H_	Ingestion rate of parasitic worms	1parasiteday^−1^	Assumed
*ρ*	Vaccine wane rate	0.7 dimensionless	[17]
*τ*_1_	Natural recovery rate for helminth-infected individuals	1/28day^−1^	
			[18]
*d*_H_	Helminth disease-induced death rate	35/1000day^−1^	
			[14]
*γ*_2_	Loss of temporary immunity for Mtb-recovered individuals	0.3day^−1^	
			[19]
*τ*_2_	Natural recovery rate for Mtb-infected individuals	0.2/365day^−1^	
			[20]
*d*_T_	Mtb disease-induced death rate	0.08day^−1^	[17]
*d*_HT_	Helminth-Mtb disease-induced death rate	0.08day^−1^	
			Assumed
*k*	Progression to active TB	0.00013/365day^−1^	[21]
*μ*_*M*_	Clearance rate of parasitic worms	13/37500day^−1^	[14]
*ε*_1_	Shading rate for helminth-infected individuals	0.09day^−1^	
			[18]
*K*	Number of parasites in the environment	10^5^ parasites	[18]
*ε*_2_	Shading rate for coinfected individuals	0.1day^−1^	Assumed
*g*	Modification parameter	1.12 dimensionless	Assumed
*σ*	Modification parameter	1.5 dimensionless	Assumed

The article "Modeling the Effects of Helminth Infection on the Transmission Dynamics of Mycobacterium tuberculosis under Optimal Control Strategies" was published in 2020. Journal: Comput Math Methods Med.

**Table 2:** Sensitivity indices for the reproduction number of Mtb infection *ℛ*_T_.

Parameter	Description	Sensitivity indices
*β*_T_	Transmission rate for Mtb	+1.0000
*k*	Progression to active TB	+0.9935
*η*	Rate of vaccination	-0.5385
*ρ*	Vaccine wane rate	+0.5385
*b*	Natural birth rate	-0.9942
*d*_T_	Mtb disease-induced death rate	-0.9691
*τ*_2_	Natural recovery rate for Mtb-infected individuals	-0.0303

**Table 3:** Sensitivity indices for the reproduction number of helminth infection *ℛ*_H_.

Parameter	Description	Sensitivity indices
*β*_H_	Ingestion rate of parasitic worms	+1
*ε*_1_	Shading rate for helminth-infected individuals	+0.4402
*μ*_*M*_	Clearance rate of parasitic worms	-1.0000
*b*	Natural birth rate	-0.0003
*d*_H_	Helminth disease-induced death rate	-0.2177
*τ*_1_	Natural recovery rate for helminth-infected individuals	-0.2221

## Data Availability

The data are available inside the manuscript, and there is no restriction on the availability of the data.

## Supplementary Materials

Supplementary Materials The supplementary material related to this article comprises the MATLAB codes used for numerical simulations.
